# Ethnobotanical inventory and medicinal perspectives of herbal flora of Shiwalik mountainous range of District Bhimber, Azad Jammu and Kashmir, Pakistan

This article has been retracted.

**DOI:** 10.1371/journal.pone.0265028

**Published:** 2022-03-29

**Authors:** Muhammad Ishtiaq, Humaira Khanum, Iqbal Hussain, Abida Parveen, Mehwish Maqbool, Sumaira Thind, Tanveer Hussain, Muhammad Azeem, Farah Shabir, Hosam O. Elansary

**Affiliations:** 1 Department of Botany, Mirpur University of Science & Technology (MUST), Mirpur (AJK), Pakistan; 2 Department of Botany, Government College University Faisalabad, Faisalabad, Pakistan; 3 Department of Biology, College of Science, University of Bahrain, Zallaq, Bahrain; 4 Department of Botany, Government Associate College for Women Layyah, Layyah, Pakistan; 5 Plant Production Department, College of Food and Agriculture Sciences, King Saud University, Riyadh, Saudi Arabia; University of Poonch Rawalakot, PAKISTAN

## Abstract

The present study was carried out to document traditional ethnobotanical knowledge (TEK) of herbal flora of District Bhimber, Azad Jammu and Kashmir (AJK), Pakistan to explore medicinal potential of wild indigenous plants (WIPs) for drug discovery. The research data was conducted during years 2015–2017 using questionnaire proforma employing structured and semi-structured interview models. The informants belonged from indigenous communities comprising of both genders with age ranging from 35–105 years. The interviews were conducted using local translator or guide who knew the dialects of all local languages. The study produced ethnobotanical inventory of 173 herbal species belonging to 45 families and out of these Poaceae was dominant family with 27 species. It was explored that maximum herbal species depicted multi-usage especially food, fodder and fuel. Among 173 herbal plant species, 69% species were used as fodder, 72% species as fuel source, 9.8% as ethnoveterinary medicines, 16% for home construction, 12% for cosmetics, 5.2% as honeybee plants and 2.7% were used as fiber source by the local people. Many local plants have been in promulgation for cure of different diseases in traditional cultures such as for cure of stomach problems, cough, cancer, jaundice, kidney diseases, diabetes, snake biting and tooth problems. Different parts of plants such as leaf, root, stem bark, flower, seed and gums are used for the treatment of different diseases by the local people. The major aliments being cured are classified into 12 disease categories by using informant consensus factor (ICF) protocol. According to ICF, the highest numbers of plant species were used against wound healing, snake bite, skin diseases, eye diseases and asthma. Fidelity level (FL) was assessed to check the reliability and use consistency of herbal drugs by the indigenous communities of the study area. The use value index (UVI) of different herb species ranged from 0.29 to 0.57 while the highest value was calculated for *Alternanthera pungens* L. (UVI: 0.57). Relative frequency of citation (RFC) value was calculated on the bases of the response of the interviewees recorded during survey in correlation with authenticating of traditional data. The RFC values represented the relative popularity of individual species in study area according to their use values. The highest value was calculated for *Alternanthera pungens* L. (0.90) and followed by *Achyranthes aspera* L. (0.80. The study reveals that many species are known for commonly used in traditional ethnomedicines (TEMs). Due to different biotic and abiotic factors in conjunction with climatic changes many herbal flora of Shiwalik mountain range (SMR) of District Bhimber of AJK is under threat. The factors like habitat loss, overgrazing, construction of communication infrastructure, silviculture practices, shelter construction (houses) and other more domestic use of wild land by clearing wild lands are boosting towards plant biodiversity loss. There is dare need to work on comprehensive exploration of TEMs to discover neo drugs from wild indigenous plants and do work for conservation of wild flora of the area for future generations.

## Introduction

Plant resources provide all necessary life sustenance materials like food, fodder, feed, forage, shelter, medicines and aesthetic values for people an area [1]. It is worth to state that a little work has been conducted on determination of conservation status of wild flora of many areas of the world. Old people or herbalists (hakims) are connected with medicinal plants and use different herbs for preparing medicines which are promulgated in the society [2, 3]. Indigenous people of rural areas of the world are primarily dependent on wild resources for fulfilling their daily life requirements. Plants play a central role in the chief health care services to the inhabitant of the area. They provide healing agents and significant raw materials to built-up of old and new medicines of homeopathic and allopathic form [3, 4]. About 80% world population depends on plants for health issues and to treat different infirmities. Herbal flora plays pivotal role in provision of nutritive and food subsistence to the dwellers of the mountains and rural areas of the world. The herbaceous plants are also key source of fodder and forage for the domesticated animals and rodents as well as for wild fauna.

Azad Jammu and Kashmir (AJK) area is rich in floral diversity because of the diverse habitats, such as streams, rivers, meadows, lakes, springs, waste lands, slopes, cultivated fields, etc. The present study was designed to study the floristic and ethnobotanical uses of herbal flora by indigenous communities of Shiwalik mountaineous range (SMR) of District Bhimber Azad Jammu and Kashmir, Pakistan (Fig 1). The study area falls in District Bhimber which was declared as an independent District in year 1996 with an area is 1516 Km^2^.

**Fig 1:** Map of study of Shiwalik mountaineous range of District Bhimber of Azad Jammu and Kashmir, Pakistan.

This area is also called as ‘Gateway to Kashmir (Bab-e-Kashmir), as Mughal emperors and warriors entered through this region to Kashmir valley and subcontinent [3, 5]. Geographically Bhimber valley is situated on 32°58’11"N Latitude and 74°4’11"E longitudes with its edaphalogical conjunction with Gujrat, Jhelum areas of Punjab province and west side with KPK province of Pakistan while on north and east side different areas of Indian occupied Kashmir [3, 6]. The rationale of the study was based on fact that “study comprises of mountains chain known as Shiwalik mountain range (SMR) which has rich phytodiversity and indigenous people of the area primarily depend wild plants and fauna resources for life sustenance. This area is yet to explore and this first time study conducted with a hypothesis that “the ethnobotanical study will assist in documentation and preservation of traditional culture of different ethnic tribes and exploration of novel botanic drug uses from medicinal plants of the area”. The pivotal key objectives of the study were multifarious comprising of (i) document floristic and ethnobotanical inventory of wild herbal flora of SMR area, (ii) to prepare data of important traditional ethnomedicines (TEMs) and enlist their botanic recipes and (iii) to determine conservation status of different plants and recommend different propagation methods.

## Materials and methodologies

### Study area

The study area comprises of hilly terrains of Shiwalik mountain range (SMR) of District Bhimber of AJK with a diverse topography (plains and hills) and phytogeography (diverse phytodiversity). The District Bhimber has mostly acidic and sandy-clay soil in nature with arid climate receiving scarce rainfall spells. Higher rainfall is recorded in July and August and lower in winter season. The average maximum and minimum temperature are 28.9°C and 15.8°C, respectively. The total average rainfall is about 1233 mm per year [7]. Average rainfall is 102.8mm per month. The area has temperature range between 0°C to 40°C with summer is bit hotter while at high altitude and forest zones the ranges preferably remains cool and low [8].

### Ethnic groups and languages spoken

The study has rich culture and ethnic groups which include “Jats, Rajpoot, Mirza, Bhatti, Moghals, Awans, Malik, Arayain, Cheema, Naramay, Kahsmiri bhatt, and Gujars”. The lingua franca spoken are “Kashmiri, Punjabi, Saraikee, Gojri, Parhayee, Urdu, Arabic and English [3, 7].

### Protocols used for data collection

In this part of research, data was collected using semi-structured and structured interview protocols following standard procedure which will consist of questionnaire and field plant interview technique [3, 9]. Many planned field trips were arranged and the area was visited with assistance of women guide or translator who was very useful to collect data from female communities of villages of SMR area of Bhimber. The interviewees were between age of 35 to 105 years comprises of both genders with diverse professions people but most were peasants and wood cutters. During Interviews using a questionnaire method to document the ethnobotanical knowledge on the herbal plant quantities, resources and their utilization by the farmers, elder people usually with the age of more than 70 years, drug dealers, hakims, shopkeepers etc. Plants were grouped on the basis of their fodder, honey bee plants, ethnoveterinary medicines, fuel and ornamental etc. The plant specimens collected, pressed, dried, preserved and were arranged alphabetically by family name, flowering period and vernacular name. The collected specimens were identified by comparing with floristic literature [10–13]) and online data comparison (www.theplantlist.org and www.eflora.org), following procedure of previous researcher [14].

### Ethical statement

The permission for field study and collection of wild plants (herbs) from wild forest areas of Shiwalik Mountian Range (SMR) zones of District Bhimber (AJK) was obtained from Departmental ethical committee (DEC) on official letter (Ref No: 31/DEC/BOT/2015; Date: 20/06/2015) and counter signed by /Head of Department. For data collection from indigenous informants, a prior verbal permission was obtained from each family head/elder man and village leader. It as acknowledged that perosnal information of each interviewee will be kept confidential as per advice and rule of DEC.

### Field survey permission letter

An official field permit (Ref No: DFO/655/2015 Dated: 01/07/2015) was obtained from District Forest Officer (DFO) to make field visits of forest area of SMR, DistrictBhimber of AJK and to collect herbal samples of plants. The right of obedience of forest rules was fully followed as per SOPs provided by the relevant office and guidance of DEC was also fully obeyed.

### Quantitative ethnobotanical tools

Ethnobotanical (EB) data collected through questionnaire method was tabulated and analyzed using quantitative analytical tools to confirm its reliability and authenticity. Several statistical tools were used for concentrating data regarding EB from study area following procedure of Amjad *et al*., 2017 and Ishtiaq *et al*., 2021 [3, 15]. For analysis of indigenous knowledge gathered from study area and its authentication was confirmed by using micro statistical tools like: “informant consensus factor” (ICF), “relative importance of plant” (RIP), “fidelity level” (FL), and “rank order of priority” (ROP) following the procedures of previous researchers like Ishtiaq *et al*., (2021) [3] and these quantitative ethnobotanical indices were prevalently utilized by previous researchers [16–18].

#### Informant Consensus Factor (ICF)

The data collected from the respondents regarding the use of various plant species were legitimated and verified by using a tool named informant consensus factor (ICF). ICF was calculated from gathered questionnaire data by using following equation;

$$ICF=\frac{Nur-Nt}{Nur-1}$$

where, Nur represents number of use citations minus (-) Nt total number of plant species used cited by respondents; divided (/) by the number of use citations in each category minus one as per given formula above. If the result is nearer to (1) or exactly (1) then reported plant species is abundantly used by locals in the area. Whereas, if value is near to (0) or comes out to be zero then reported plant species is casually used by inhabitants of area [19].

#### Fidelity Level (FL)

The fidelity level of the data was calculated which depicts the percentage (%age) of interviewees claiming any use of a particular plant for the same major purpose or field and total number of commonly reported usages or ailments. It was calculated according to formula:

$$FL=\frac{Np}{N}\;x\;100\;(\%)$$

Whereas; Np depicts number of informants, who claimed a particular use of a plant species used for a typical disease and N means that number of informants/interviewees who used the plants as an ethnomedicine to treat given diseases [3, 20].

#### Rank Order Popularity (ROP)

To determine correction between FL and RPL rank order popularity is used. ROP designate the popularity rank to individual in accordance to FL and RPL values [3, 21]. Following formula was used for ROP calculation:

ROP=FLxRP

ROP value represents higest rank/level for popularity of various MPs used to cure specific disorder RPL and ROP statistical test are significantly important for determining EB importance of commonly used plant in respected area.

#### Relative Popularity Level (RPL)

RPL describes the frequency use of a particular species. In some analysis, sporadically FL provides same usage frequency of various species then Relative popularity level index is used to reassure and confirm FL values of various trial species. RPL value generally ranges in-between 0–1, where value 1 or nearer value to 1 represents maximum RPL value while 0 or nearer to 0 represents minimum value frequency for particular disease [3, 22]. Value of RPL increases in accordance with informants as it rises correlation coefficient factor r = 0.10. For example, if a particular species is reported by 25 or more individuals it will have high RPL value and vice versa. RPL is calculated by proportion of (I_u_ /number of individuals reported the use of particular plant). When 25 of more individuals report for a particular species RPL value becomes (I_u_/12) which gives one (1) and species is ranked as Popular (P). Whereas if less than 25 individuals report plants uses then respected plant species is ranked as unpopular (UP) as stated by Ishtiaq *et al*., [23, 24]. Marginal value in-between, P and UP of particular plant refers point where further increase in number of informants don’t upswing medicinal use per plant species.

#### Relative Importance of Plant (RIP)

To determine the pharmacological or pharmaceutical significance of individual plant relative importance of plants (RIP) was used following protocol of Umair and Amjad [25].

$$\mathrm{RIP}=\frac{\mathrm{Rel}.\;\mathrm{Ph}+\mathrm{Rel}.\;B.S.}{2}\times 100$$

whereas Ph. is pharmacological features of the plants and Rel. Ph: relative pharmacological importance; rel. BS: body system treated. The relative Pharmacological significance can be caluclated by the given below formula.

$$\mathrm{rel}.\;\mathrm{Ph}.=\frac{\mathrm{Ph}.\;\mathrm{of}\;\mathrm{given}\;\mathrm{Plant}}{\mathrm{Ph}\;\mathrm{of}\;\mathrm{all}\;\mathrm{reported}\;\mathrm{plant}\;\mathrm{species}}$$

whereas Ph. is pharmacological attributes of the each provided plant and rel. Ph. is the relative number of pharmacological properties referenced for an individual plant.

$$\mathrm{rel}.\mathrm{BS}=\frac{\mathrm{BS}\;\mathrm{of}\;\mathrm{given}\;\mathrm{Plant}}{\mathrm{BS}\;\mathrm{of}\;\mathrm{all}\;\mathrm{reported}\;\mathrm{plant}\;\mathrm{species}}$$

where BS is the number of body System healed by single plant species whereas, rel. BS is total relative number of body system treated by the given plant species.

#### Use value index

The use value index (UVI) demarcates relative importance of different uses of the specific species. It was determined by using past cited formula following protocol of Long *et al*., 2013 and Leto *et al*., 2013 [26, 27].


$$UV_{i}=\frac{\sum Ui}{N}$$

Whereas UV indicates “relative use value” of the single species; “U” is the ‘number of uses mentioned by each informant for the species and “N” is the ‘total number of informants who reported that species.

#### Relative Frequency of Citation (RFC)

Relative frequency of citation is used an index to explore significance or importance of each species occurring in the local area. RFC was determined by “dividing the number of informants” confirming the frequency.


$$RCF=\frac{FC}{N}R$$

Where, ‘0 < RFC >1’; and FC is the ‘number of informants’ reporting use of a particular species and N is the ‘total number of informants’ involved in study survey.

#### Priority Ranking (PR)

Priority ranking (PR) method was used for indicating the preference of the local people about the potential use of each plant in certain use and it describes the biotic pressure on the plants of the area and it assists to calculate the conservation status of various species in the study area [28, 29].

## Results and discussion

The research work was carried out in District Bhimber during years 2015–2107 prevalently based on SMR areas of AJK, Pakistan. The plants samples free of disease were collected, pressed, dried in newspapers and mounted as per standard herbarium protocol of Ishtiaq *et al*., (2021) [3]. These specimens were mounted on herbarium sheets, then identified, preserved and deposited in Herbarium of Mirpur University of Science and Technology Bhimber Campus, AJK. In the investigated area 173 herbaceous plant species belonging to 45 families were found and recorded for EB and TEMs data. Among 45 families Poaceae were the dominant families with 27 species. There were followed by Papilionaceae, Amaranthaceae and Fabaceae with 8 and 7, 7 species, respectively. These were followed by Boraginaceae and Lamiaceae with 06 species, Cyperaceae 05 species each, Chenopodiaceae, Euphorbiaceae, Plantaginaceae, Ranunculaceae and Solanaceae 04 species each and Acanthaceae, Liliaceae, Malvaceae, Brassicaceae, Cucurbitaceae, Portulaceae, Papaveraceae 03 species each (Table 1). Similar results were explored and published by Ajaib *et al*., 2014 in District Kotli, Azad Jammu and Kashmir [30]. Plant is an unusual organism of infinite kindness and compassion it offers to mankind, the creation of its life activities in different ways. Among them domestic, commercial and industrial uses are well known.

**Table 1:** Family index of herbal flora of District Bhimber of AJK Pakistan.

Sr. No.	Families	No. of species	Sr. No.	Families	No. of species
01.	Amaranthaceae	7	24.	Fabaceae	7
02.	Alliaceae	1	25.	Lamiaceae	6
03.	Aizoaceae	1	26.	Liliaceae	3
04.	Adiantaceae	2	27.	Leguminosae	1
05.	Aristolochiaceae	1	28.	Labiatae	2
06.	Asclepiadaceae	1	29.	Malvaceae	3
07.	Acanthaceae	3	30.	Nyctaginaceae	1
08.	Berberidaceae	1	31.	Oxalidaceae	1
09.	Boraginaceae	6	32	Poaceae	27
10.	Brassicaceae	3	33.	Phyllanthaceae	1
11.	Caryophyllaceae	1	34.	Portulacaceae	3
12.	Chenopodiaceae	4	35.	Papaveraceae	3
13.	Cyperaceae	5	36.	Papilionaceae	8
14.	Convolvulaceae	1	37.	Phyllanthaceae	1
15.	Cucurbitaceae	3	38.	Papilionaceae	2
16.	Crassulaceae	1	39.	Plantaginaceae	4
17.	Caesalpiniaceae	2	40.	Primulaceae	2
18.	Celastraceae	1	41.	Ranunculaceae	4
19.	Cactaceae	1	42.	Rubiaceae	2
20.	Cuscutaceae	1	43.	Solanaceae	4
21.	Equisetaceae	1	44.	Verbenaceae	2
22.	Euphorbiaceae	4	45.	Zygophyllaceae	1
23.	Fumariaceae	1			

### Ethnobotanical findings

Ethnobotany includes all aspects of traditional uses of plants including food, poison, fodder, timber, clothing, dyes, fuel, medicines and veterinary medicines. Ethnobotanical survey of SMR region of District Bhimber gave evaluation of relation between man and his surrounding plants. For this purpose, many field surveys were carried out in the certain selected sites of the study area of SMR. Many ethnobotanical plant species were recognized along with data about traditional uses and villagers of the area. Among 173 herbal plant species, 69% species were used as fodder, 72% species were used for fuel purpose, 9.8% were used as ethnoveterinary purposes, 2.7% were used as fiber, 5.2% were used as honeybee plants, 16% were used as domestic and 12% were used as cosmetics (Table 2 and Fig 2). Similar studies were also conducted by Hussain *et al*., 2012 when they studied the ethnobotany of plants (Angiosperm) flora of Rawalakot. They represented 173 medicinal plants used by native people for different purposes and cure of human and livestock. About 111 species are weeds, 158 used for fodder, 68 species used as fuel, 33 species were fruit yielding 22 were used as timber, 31 as ornamental, 25 as fencing lawns and fields. While 21 species were used as vegetables, 9 for thatching houses and huts; and 13 species were recorded as poisonous. Shaukat *et al*., (2012), studied ethnobotanical studies of diversity of plants of some selected regions of Rawalakot [31]. They concluded that 26 plant species belonging to 19 families were used by local people for different purposes. Sedges and grasses of the study area were grazed as fodder by animals in Summer and Spring seasons and stored for Winter and Autumn when no fodder is accessible for grazing. The relationship between plants and people is extraordinary because plants provide fodder, domestic animals, food, ethno veterinary, fuel and honeybee, flowers for esthetics and happiness [30, 32]. It was studied that due to grazing off domestic animals in the hilly areas of District Bhimber and over harvesting of every available portion of the gainful medicinal plants by indigenous communities as a source of income creates severe plethora of biotic pressure leading towards loss or extinction in future. Generally, women were mostly linked with collection of herbal plants as source of botanic drugs who collect and dry these phyto-drugs at home, on rocks or on mats, then after sprinkling the plants on roof. The dried collected herbal plants were sold directly to the main city markets and provincial drug traders. Similar results were also shown by Khan *et al*., (2011) during whose work conducted on the ethnomedicinal evaluation of plants of Hindu-Kush area of Pakistan [33].

**Fig 2:** Ethnomedicinal uses of herbs of Shiwalik Mountain Range of District Bhimber of AJK Pakistan.

**Table 2:** Ethnobotanical uses of plants (%age) from Shiwalik mountain range of District Bhimber of Azad Jammu and Kashmir, Pakistan.

Sr. No.	Ethnobotanical Uses	%age
01	Fodder	69
02	Fuel	72
04	Fiber	2.7
05	Cosmetics	12
06	Domestic	16
07	Ethnoveterinary	9.8
08	Honey bee plants	5.2

### Ethnomedicinal uses

Among173 herbaceous plants, belonging to 12 families, 21.4% species used against skin diseases followed by 16.7% used for wound healing and 14.4% used against fever. These were followed by 17.3% for stomach problems, 12.13% for cough and 22.7% for treatment of cancer. The study revealed that17.14% species were used against jaundice, 4.6% were used against asthma and 8.09% for kidney diseases. These were followed 9.2% of herbal flora which was used for diabetes, 4.62% against snake biting and 1.7% species were used for treatment of tooth problems (Tables 3 and 4; Fig 2). Similar results were also shown by Shinwari, (2000) who carried out his research on Margalla Hills, National Park [34]. Another researcher, Ahmad, 2007 highlighted and demarcated the medicinal plants around motorway Pakistan with their potential for neo-drug discovery. Sheikh, *et al*. 2002 studied ethno botanical and ethnomedicinal uses of wild plants of Naltar valley of Karakorum, Pakistan [35]. Similar, studies were also conducted by Shinwari *et al*., 2010 and Farooq *et al*., 2012 who demonstrated that local people of village areas depend on wild indigenous plants (WIPs) [36, 37]. These findings confirmed that ‘diabetes, anticancer and skin diseases were the most commonly occurring diseases in the area that is due to extreme use of ghee (solidified oil/butter refined form) and change of life style towards comfortable mode. Similar studies were conducted by Hussain *et al*., (2012) who depicted that change of life style towards sedentary and luxurious form was cause of many acute and chronic infirmities [38]. They concluded that 59 medicinal plants are frequent used by the local people of Rawalakot for themselves out of 173 medicinal plants for cure of different ailments. The frequently used medicinal plants are *Mentha longifolia*, *Achyranthes aspera*, *Podophyllum emodi*, *Valeriana jatamansi*, *Berberis lycium*, *Punica granatum*, *Achillea millefolium*, *Aesculus indica*, *Amaranthus viridis*, *Viola odorata*, *B*.*stracheyi*, *Cichorium intybus*, *Elaeagnus umbellate*, *Ficus palmate*, *Funiculus vulgare*, *Zanthoxylum erratum*, *Plantago major*, *Bergenia ciliate and Melia azedarach*. Our findings are also coincided with the previous cited works of the above stated authors.

**Table 3:** Percentage of plant species used for treatment of different diseases from Shiwalik mountain range of District Bhimber of Azad Jammu and Kashmir, Pakistan.

S. No.	Disease categories	%age of plant species	S. No.	Disease Categories	%age of plant species
01.	Skin diseases	21.9	07.	Jaundice	17.14
02.	Wound healing	16.7	08.	Asthma	4.6
03.	Fever	14.4	09.	Tooth problems	1.7
04.	Stomach diseases	17.3	10.	Kidney diseases	8.09
05.	Cough curing	12.13	11.	Diabetes	9.2
06.	Cancer	22.7	12.	Snake biting	4.62

**Table 4:** Ethnomedicinal uses of herbaceous plants from Shiwalik mountain range of District Bhimber of Azad Jammu and Kashmir, Pakistan.

Sr. No.	Botanical Name of Plant	Common Name	Family	Part used	Traditional Ethnomedicinal uses
01.	*Achyranthes aspera* L.	Phothkanda	Amaranthaceae	Fruit	Fruits are roosted, grinded and used against asthma, fever, cough and constipation.
	MUH-1681				
02	*Astragalus leucocephalus* Benth.	Kathi	Fabaceae	Leaf	Powder of leaf is used to cure stomach pain, gastrointestinal pain and kidney diseases.
	MUH-1678				
03.	*Amaranthus viridis* L. MUH-1682	Ganar	Amaranthaceae	Whole plant	Plant is taken dried, make powder and used with water to cure sore boils bleeding, diarrhea and wound healing.
04.	*Amaranthus tricolor* L. MUH-1683	Bhaji	Amaranthaceae	Leaf, root	Extract of leaf is used as effective tonic for cure of snake bite, diuretic and wound healing.
05.	*Achyranthes bidentata* L. MUH-1684	Phothkanda	Amaranthaceae	Whole plant	Ethanolic extract of leaf is used for healing wounds, diuretic, treat cancer, eye related diseases and anemia.
06.	*Aerva javanica* (Burm.f.) Juss.	Bui	Amaranthaceae	Whole plant	Extract of plant used to cure different diseases like diarrhea, microbial infections and cure kidney diseases.
	MUH-1685				
07.	*Anagallis arvensis* L. MUH-1686	Bili booti	Primulaceae	Leaf	Leaf extract is used to treat stomach diseases, antifungal and wound healing.
08.	*Abutilon indicum* L.	Sweet kangi	Malvaceae	Whole plant	Paste of seeds and lea is used to cure skin diseases. Aerial parts are used to cure asthma, diarrhea, cancer, inflammatory and diabetic
	MUH-1687				
09.	*Aerva sanguinolenta* (L.)Blume.	Chiti boti	Amaranthaceae	Whole plant	Extract of plant used to cure different diseases anti-diarrheal, antimicrobial and cure kidney diseases.
	MUST-1688				
10.	*Alternanthera pungens* L. MUH-1689	Taahee booti	Amaranthaceae	Whole plant	Ethanolic extract of leaf is used for healing wounds, diuretic, treat cancer, eye related diseases and anemia.
11.	*Argemone mexicana* L. MUH-1690	Dudhli	Papaveraceae	Whole plant	Extract of whole plant is used to treat different diseases like wound healing, -inflammation, bacterial infection, diuretic, cancer and tumors.
		kandyari			
12.	*Artemisia scoparia* Waldst. & Kit.	Red stem	Asteraceae	Leaf, flowers	Leaves are dried and made paste which is used with water to cure stomach diseases and intestinal worms and relevant diseases.
	MUH-1691				
13.	*Allium Jacquemontii* Knuth. MUH-1692	Jangli piaz	Alliaceae	Blub, leaf	Juice of plant parts is used to treat different disease like snake bite, scorpion bite and microbial infections.
14.	*Aloe vera* L.	Kawar gandal	Liliaceae	Leaf	Leaf pulp is applied on wounds for healing and pulp is mixed with sugar used against cardiovascular diseases, cancer, diabetes and neurological infirmities.
	MUH-1693				
15.	*Avena fatua* L.	Wild oat	Poaceae	Seeds	Seeds are grinded and its powder is used for curing diseases of skin, nails and muscles. It is also very effective in cardiovascular diseases.
	MUH-1695				
16.	*Acrachne racemosa* L.	Goose grass	Poaceae	Whole plant	The plant is used fodder for animals. Its paste of root is used for curing infirmities of skin, wounds, kidney disorder and breathing issues.
	MUH-1696				
17.	*Aristolochia punjabensis* Lace. MUH-1697	Pipevine	Aristolochiaceae	Roots	Powder of root is taken with milk to treat body pain. The root powder is used with water to cure menstrual problems, body pain and vaginal infections.
18.	*Adiantum capillus-veneris* L. MUH-1698	Median hair fern	Adiantaceae	Whole plant	Whole plant is dried, powdered and its small amount is used for lowering blood pressure, curing cough, fever, hypertension and hair caring.
19.	*Adiantum incisum* L. MUH-1699	Fern	Adiantaceae	Leaf	Infusion of leaves is used for cough and other diseases like fever and body weakness.
20.	*Asplenium trichomanes* L.MUH-1700	Bird nest fern	Caesalpiniaceae	Leaf	Leaf is smoked for chest pain, colds, headache, cure colds and chest pain.
21.	*Asphodelus tenuifolius* Caven. MUH-1701	Bhokal	Liliaceae	Seeds	Seed powder is taken in piles and used to cure other skin diseases.
22.	*Ajuga bracteosa*	Hari booti	Lamiaceae	Whole plant	Whole plant is effective for curing pimple and boils diseases. Root powder is used to cure diarrhea. Leaf powder is used to cure malarial fever, cure stomach diseases, diabetes and dysentery.
	Benth.				
	MUH-1702				
23.	*Aristida adscensionsis* L. MUH-1703	Saroot	Poaceae		The whole plant is used as fodder for animal and rodents. The root decoction is used for cure of skin allergy.
24.	*Berberis lyceum* L. MUH-1708	Sumblu	Berberidaceae	Bark	Powder of bark is applied on wounds for healing, diabetes, skin allergies, scabies jaundice and piles.
25.	*Boerhavia diffusa* L. MUH-1709	Sanati	Nyctaginaceae	Roots, leaf	Roots re crushed and boiled in milk which is used to remove kidney stones. Root decoction is used for treating pneumonia, abscesses and jaundice. The root are cut into pieces and its garlic is used for relief of hepatitis and jaundice in rural areas.
26.	*Buglossoides arvensis* L. MUH-1711	Kalu	Boraginaceae	Leaf	Infusion of leaves are sedative. The leaf powder is used for stomachache.
27.	*Barleria cristata* L.	-	Acanthaceae	Root, leaf, seeds	Bitter juice used to treat diseases like lung disorders, snake bite, microbial infections, diabetes and toothache.
	MUH-1712				
28.	*Bryophyllum pinnatum*	Pather chatt	Crassulaceae	Leaf	Fresh leaves are warmed and rapped on pains of knees and also used for wound healing by local rural people.
	L. MUH-1713				
29.	*Bromus japonicus* L. MUH-1714	Broom grass	Poaceae	Whole plant	Powder of whole plant is used to treat different disease like chest pain, anti-inflammatory and hepatitis.
30.	*Cannabis sativa* L.	Bhang	Cannabaceae	Leaf	Leaf paste is used for wound healing. Leaves are used as narcotics so used to generate pleasant, cure cough, headache, abdominal pain, used for pleasant and excitement. It is also used for cure of sleep disorders and anxiety. The extract of leaf is used for treatment of epilepsy.
	MUH-1719				
31.	*Capparis sepiaria* L.	Kareer	Cyperaceae	Whole plant	Decoction of whole plant is used to treat disease like antimicrobial, antifungal and skin diseases.
	MUH-1720				
32.	*Calendula arvensis* L. MUH-1721	Field marigold	Asteraceae	Leaf and flowers	Extract of leaves is used to cure antiseptic, cure skin diseases and healing of wounds.
33.	*Carthamus lanatus* L. MUH-1722	Distaff thistle	Asteraceae	Flowers, seeds	The paste of seeds is prepared and applied to cure different skin diseases and fever. The flower decoction is used to fever and chest cold feelings.
34.	*Calendula officinalis* L. MUH-1723	Marigold	Asteraceae	Leaf, flowers	The sap of flowers used to cure skin diseases and treatment of cancer. The external use of plant in form of extract with tincture is effective for wound healing, blood purifier, cure skin disorders, anticancer, anemia and kidney diseases
35.	*Carthamus oxyacantha* L.	Kandyari	Asteraceae	Flowers, seeds	Flowers are used to cure jaundice while oil extracted from seeds is used to cure skin diseases and cure jaundice.
	MUH-1724				
36.	*Chenopodium ambrosioides* L.	Mexicana tea	Chenopodiaceae	Leaves, flowers, and seeds.	Dried leaves are used to treat cancer. Seed oil is used to cure arthritis and skin diseases.
	MUH-1725				
37.	*Chenopodium botrys* L. MUH-1726	Oak	Chenopodiaceae	Leaves and seeds	Fresh leaves extract is used to cure kidney diseases, arthritis, skin diseases, digestive, cough and pectoral pains.
38.	*Chenopodium album* L. MUH-1727	Bathu	Chenopodiaceae	Leaves	Leaf juice is used to cure kidney problems and cure spleen enlargement problems.
39.	*Colebrookea*	Bansa	Labiatae	Leaf, root, bark	Powder of plant parts is used to treat different diseases like cure flu, fever, wound healing and epilepsy.
	*Oppositifolia* Smith.				
	MUH-1728				
40.	*Ceropegia bulbosa* L.	Galot	Asclepiadaceae	Tuber,	Juice of plant parts is used to treat diseases like cancer, microbial infectious diseases, kidney disorders, digestive problem.
	MUH-1729				
				Leaves	
41.	*Convolvulus arvensis* L. MUH-1730	Rawari	Convolvulaceae	Whole plant	Dried powder of plant mixed with gurr (dired juice of sugar cane) to treat constipation. Leaf paste is used to cure skin diseases, cure constipation and anti-inflammation.
42.	*Cichorium intybus* L. MUH-1731	Kasni	Asteraceae	Seeds, leaves	Powder of seed is used to treat different diseases like fever, kidney problems, vomiting, toothache and blood purifier
43.	*Chenopodium*	Gandi	Chenopodiaceae	Leaf, root	Paste and juice of plant parts is used to treat different diseases like wound healing, constipation, skin burns and stomach pains.
	*ambrosioides* L.	booti			
	MUH-1732				
44.	*Cuscuta reflexa* Roxb.	Neel dhari	Cuscutaceae	Whole plant	Whole plant extract is used to treat viral diseases, juice is used to cure jaundice, warm paste is used to treat headache. The decoction is used to treat cough, arthritis, skin disorders and blood purifiers.
	MUH-1733				
45.	*Cynodon dactyolon*	Khabal	Poaceae	Whole plant	Paste of fresh plant is applied on wound healing, skin diseases and fever. It is also used as diuretic and cure of inflammations.
	L. MUH-1734				
46.	*Cenchrus ciliaris*	Ghass	Poaceae	Whole plant	Plant is crushed and made powder and used for curing different diseases like kidney diseases, tumors and wound healing
	L. MUH-1735				
47.	*Cynoglossum lanceolatum* Forrsk.	Leendra	Boraginaceae	Whole plant	Bark of plant is used to cure teeth diseases. Root paste is used to cure cough and tuberculosis diseases.
	MUH-1736				
48.	*Cordia obliqua* L.	Lasoora	Boraginaceae	Whole plant	Fruit of this herb is used to cure dry cough, fever and chest pain. Bark juice is used to cure tonic diseases. Leaves are also effective for headache and ulcers.
	MUH-1737				
49.	*Cassia obtusifolia* L. MUH-1738	Coffee weed	Fabaceae	Leaves, root, seed, flowers	Leaves are used to make tea to remove headache and migraine. Seed powder is used to cure vomiting, skin diseases, ulcers, asthma and eye diseases.
50.	*Cenchrus biflorus* Del MUH-1739	Gass	Poaceae	Leaves and seed	Leaf extract is used to treat different diseases, diuretic, digestive, anti-inflammatory, fever and cold.
51.	*Cortusa brotheri* L. MUH-1741	-	Primulaceae	Seed and stem	Extract of plant used to treat different diseases like stomach pain and constipation.
52.	*Cyperus esculentus* L. MUH-1742	Nut sadge	Cyperaceae	Whole plant	Extract of whole plant is used to treat different diseases. It is used as medicine i.e. anti-malarial, anti-diarrheal, antidiabetic, antioxidant and antibacterial source of medicines.
53.	*Cyperus iria* L. MUH-1743	Flat sadge	Cyperaceae	Root and fruit	Dried parts of plants are used to cure different diseases like cough, chronic, fever, cold, arthritis and cardiac diseases.
54.	*Cyperus rotundus* L. MUH-1744	Purple sadge	Cyperaceae	Root tubers	Roots are grinded, make powder and used with water. Tubers cooked are used to cure digestive and uterus pains.
55.	*Clitoria ternatea* L. MUH-1745	Butterfly pea	Fabaceae	Stem, flower, leaf, fruit	Alcohol extract of plant used to treat different diseases like mental illness, antibacterial, antidiabetic and anti-inflammatory.
56.	*Citrullus lanatus* L. MUH-1746	Cheebar	Cucurbitaceae	Seed, leaves	Dried pulp of leaves and root are used to treat different diseases like constipation, ulcers, cancer.
57.	*Citrullus colocynthis* L. MUH-1747	Tumma	Cucurbitaceae	Root and fruit	Extract of whole plant is used to treat different diseases like tumor, ulcers, remove pain and swelling.
58.	*Coronopus didymus* L. MUH-1749	Jangliu halon	Brassicaceae	Whole plant	Powder of plant is used to treat different diseases like relive pain and inflammatory.
59.	*Carissa opaca* L. MUH-1750	Amaltas	Caesalpiniaceae	Root	Powder of dried root is applied on wounds. The latex is used antiseptic for cure of foot and skin diseases. The leaf is used as fodder for rodents.
60.	*Digera muricata* L. MUH-1752	-	Poaceae	Whole plant	Infusion of plant used to treat stomach diseases, digestive disorders and urinary diseases.
61.	*Dicliptera roxburghiana* News. MUH-1755	Kali boti	Acanthaceae	Plant sap, leaves, flower	Dried parts of plants are used to treat different diseases like diuretic, skin diseases, toxic.
62.	*Dicliptera bupleuroides* News. MUH-1756	Marvel grass	Poaceae	Whole plant	Powder of plant is used treat different diseases like antidiabetic and antimicrobial
63.	*Dichanthium annulatum* Forssk. MUH-1757	Crabgrass	Poaceae	Whole plants	Dried parts of plant are used to treat different diseases like diuretic. The lead is used as laxative knowntonic for stomach issues and detoxifier of toxic materials of intestines.
64.	*Digitaria ciliaris* Retz. MUH-1758	Finger grass	Poaceae	whole plant	Fodder for animals.
65.	*Digitaria nodosa* L. MUH-1759	Grass crow foot	Poaceae	whole plant	Fodder for animal.
66.	*Equisetum arvensis* L. MUH-1764	Horsetail	Equisetaceae	Whole plant	Plant juice is used for kidney diseases. The stem decoction is used for cure of stomach issues. The renal problem is cured by its infusion.
67.	*Euphorbia hirta* L. MUH-1765	Dhodke	Euphorbiaceae	Whole plant	Its seeds are ground into powder and used with milk to cure diarrhea. The leaf decoction is used cure of chest infirmities.
68	*Euphorbias prostata* L. MUH-1766	Sand mat	Euphorbiaceae	Whole plant	Plant is crushed and eats to remove kidney stones. It is used anti-hemorrhoids.
69.	*Euphorbia helioscopia* L. MUH-1767	Cathri dodak	Euphorbiaceae	Whole plant	Powder of root is used to cure skin diseases. It is also poisonous for cattle if engulfed too much.
70.	*Euphorbia prolifera* L. MUH-1768	Dodak	Euphorbiaceae	Whole plant	Whole plant is taken in form of powder and used to cure diseases.
71.	*Eclipta prostrata* L. MUH-1769	Flase daisy	Asteraceae	Whole plant	Whole plant is taken dried make powder used to cure different diseases like hepatitis, nervous disorders, anemia, skin diseases.
72.	*Evolvulus alsinoides* L. Bioss.	Morning glory	Poaceae	Leaves	Extract of leaf is taken for constipation, vomiting and indigestion.
	MUH-1770				
73	*Echinochloa crus-galli* L.	Cockspur grass	Poaceae	Shoots, roots, seed	Seed can be cooked, sieve, bitter flavor used to prevent different diseases like stomach pains, inflammation, wound healing, cancer, sores and hemorrhages.
	MUH-1771				
74.	*Eleusine indica* L.	Goose grass	Poaceae	Whole plant	Extract of plant parts used to treat different diseases like kidney, diarrhea, eye diseases and dysentery.
	MUH-1772				
75.	*Ehretia laevis* Roxb.	Sakkar	Boraginaceae	Whole plant	Extract of different plant parts is used to treat diseases, skin cancer, anti-inflammatory and wound healing.
	MUH-1773				
76.	*Fumaria indica* L.	Papra	Fumariaceae	Whole plant	Herb is dried make powder and used to treat different diseases like diuretic, cure liver and digestive diseases and cure skin diseases.
	MUH-1780				
77.	*Galium aparine* L.	Lahndara	Rubiaceae	Whole plant	Plant is crushed make powder and used to treatment of different diseases like cure fever, diuretic, wound healing and antiseptic.
	MUH-1784				
78	*Galium elegans* L.	Jari	Rubiaceae	Whole plant	Taken whole plant dried, crushed and makes powder used with water to cure different diseases like Jaundice, antiseptic, wound healing and fever
	MUH-1785				
79.	*Gagea elegans* Wall. MUH-1786	Yellow star	Liliaceae		Fodder for animals for rodents and snow cocks.
80.	*Heteropogon contortus* L. MUH-1788	Sarala grass	Poaceae	Whole plant	It is used as fodder for cattle and rodents.
81.	*Heliotropium strigosu*m Willd. MUH-1789	Gorakh pan	Boraginaceae	Leaves, stem, root	Gum is used to treat boils. Juice for snake bite, diuretic, sore pain, wound healing and used to treat boils.
82.	*Helianthus tuberosus* L. MUH-1790	Artichoke	Asteraceae	Whole plant	Whole pant is used to treat different diseases diuretic, antidiabetics, stomach diseases, tonic effect, antidiabetic, anti-microbial.
83.	*Hyoscyamus niger* Linn.	Khoob kalan	Solanaceae	Whole plant	Powder of whole plant is used to treat different diseases like pain killer and kidney stones.
	MUH-1791				
84.	*Imperata cylindrica* L.	Grass	Poaceae	Root, flower	A decoction of the root is used to treat digestive diseases, wound healing, anti-jaundice and dysentery.
	MUH-1793				
85.	*Ipomoea eriocarpa* R.Br.	Wanweer booti	Convolvulaceae	Whole plant	Crush whole plant, make powder and extract is used to cure skin diseases and cancer.
	MUH-1794				
86.	*Kyllinga brevifolia*	-	Cyperaceae	Rhizome, leaves, tubers	Extract of plant parts used to treat different diseases like digestive, diuretic, tonic, sedative, antimalarial, snake bite.
	Rottb.				
	MUH-1799				
87.	*Loranthus longiflorus* Desr.	Purakh	Loranthaceae	Flowers, leaves	Decoction of plant is used to treat different diseases like diabetes, skin diseases, wound healing, bone repairing.
	MUH-1800				
88	*Lantana camara* L.	Panj pholi	Verbenaceae	Leaves	Ethanolic extract of leaves are reported for wound healing, Skin diseases, anticancer, anti-inflammatory, malarial diseases.
	MUH-1801				
89.	*Larotalaria medicaginea* Lam. MUH-1, 803	Rattle pods	Fabaceae	Whole plant, leaves	Make powder of whole plant and used to treat different diseases like malaria, constipation, fever
90.	*Lathyrus aphaca* L.	jangle matr	Fabaceae	Whole plant	Powder of whole plant is used to treat different diseases like burns, anti-inflammatory, anti-bacterial
	MUH-1804				
91	*Leucas aspera* L.	Thumbai	Libiateae	Whole plant	Flower are mixed with honey and used for different diseases like fever, cough, cold, ulcer
	MUH-1805				
92.	*Launaea procumbens* Roxb.	Bathala	Asteraceae	Whole plant	Powder of whole plant is used treat different diseases like skin diseases, cough, chest pain, obesity, constipation
	MUH-1806				
93.	*Maytenus royleana* Wall.	Patakee	Celastraceae	Bark, leaves	Paste of Bark and leaves used for bone fractures and other skin diseases.
	MUH-1811				
94.	*Malva parviflora* L.	Sonchal	Malvaceae	Whole plant	Leaves extract with water is used to cure different diseases, anti-inflammatory, antimicrobial
	MUH-1812				
95.	*Malva sylvestris* L.	High mallow	Malvaceae	Seeds	Seeds are boiled, add sugar made sharabt used to cure fever and cough
	MUH-1813				
96.	*Melilotus alba* L.	Shinji	Fabaceae	Leaves	Infusion of leaves is used to treat different diseases including dysentery, cough, bronchial disorders, abdominal pain
	MUH-1814				
97.	*Micromeria biflora* L.	Marathi	Leguminosae	Leaves, root	Root extract is to cure different diseases. Leaf oil used as flavoring agent, cure dysentery, colds, cough, abdominal pain
	MUH-1815				
98.	*Melilotus indica* (L.) All.	jangle	Papilionaceae	Leaves	Leaf juice is used against antibacterial disorders.
		methi			
	MUH-1816				
99.	*Medicago polymorpha*	Sriri	Papilionaceae	Whole plant	Seed can be ground into a powder and mixed with water and used to treat different diseseaes like cure skin diseases, dysentery, wound healing
	L. MUH-1817				
100.	*Mentha royleana*	Wild mint	Labiatae	Leaves, stem	Leaves are dried and, make powder used to cure different diseases like cough, throat pain, digestion and constipation.
	Benth. MUH-1818				
101.	*Nasturtium officinale*	Chooch	Brassicaceae	Leaves	Leaf juice is taken for stomach diseases, ulcers, intestinal pain
	R.Br.				
	MUH-1820				
102.	*Nicotiana plumbaginifolia* Viv. MUH-1821	Jangli tobacco	Soalnaceae	Whole plant	Powder of leaves used to treat different diseases like healing of wounds and cuts toothache, rheumatic
103.	*Otostegia limbata* L.	Kori booti	Lamiaceae	Leaves	Leaves are dried, grind and powder are applied on wound
	MUH-1822				
104.	*Oxalis corniculata* L.	Khati boti	Oxalidiaceae	Fruits and seeds	Plant sap is used to cure skin diseases. It is also used as laxative of stomach disorders.
	MUH-1823				
105.	*Ocimum bacilicum* L. MUH-1824	Naiazbu	Lamiaceae	Leaves, seeds	Leaf extract is used to cure cough. Seed powder is used in cold drinks. It is also used in headache and cough cure.
106.	*Ocimum tenuiflorum* L. MUH-1825	Tulsi	Lamiaceae	Leaves	Leaves are crushed mixed with water make juice used for treatment of different diseases like cure fever, anticancer, skin disorders, heart related diseases.
107.	*Opuntia dillenii* Haw. MUH-1826	Thor	Cactaceae	Stem	Decoction of whole plant is used orally to treat different diseases like asthma, Anti-diabetics, ulcer, Anti-inflammatory, antimicrobial
108.	*Polygonum plebeium* L. MUH-1829	-	Polygonaceae	Whole plant	Extract of plant is used to treat different diseases like pneumonia, liver diseases, heart related disease
109.	*Persicaria barbata* L. MUH-1830	Jor booti	Polygonaceae	Whole plant	Extract of whole plant is used to treat different diseases like kidney stones, ulcers, asthma, sedatives, gastric diseases, insecticides.
110.	*Parthenium hysterophorus* L. MUH-1835	-	Asteraceae	Whole plant	Extract of whole plant is used treat different diseases, anticancer, antidiabetic. It is also used in neralgia and malaria.
111.	*Plantago lanceolata* L. MUH-1836	-	Plantaginaceae	Leaves	Take leaves of plant make paste and applied on inflamed places.
112.	*Prosopis farcta* L.C. VC. HB. MUH-1837	-	Plantaginaceae	Bark, flowers	The flowers are mixed with sugar and use to prevent miscarriage. Bark is effective for different diseases like asthma, dysentery, skin diseases, snake bite.
113.	*Papaver dubium* L.	Jungle post	Papaveraceae	Flowers, stem	Infusion of whole plant is used to treat different diseases like cough, fever, antimicrobial
	MUH-1838				
114.	*Panicum turgidum* Forssk MUH-1839	-	Poaceae	Whole plant	Extract of whole plant is used to treat different diseases like wound healing, throat infection, smallpox
115.	*Pennisetum flaccidum* Griseb. MUH-1840	Fountain grass	Poaceae	Whole plant	Plant parts is used to treat different diseases like fever
116.	*Phragmitis karka* (Retz.)MUH-1841	Babyoon	Poaceae	Whole plant	Roots are cooling and used as antidiabetic. It is used as analgesic. Cure of depressant and hyperglycemic effect.
117.	*Poa annua* L.	Grass	Poaceae	Leaves	Whole plant is used as fodder
	MUH-1842				
118.	*Phalaris minor* L.	Bunch grass	Poaceae	Leaves, fruit, seed	Leaves are dried and made Joshanda (admixture) is used to cure cough, cold and other diseases like dysentery, fever, diarrhea.
	MUH-1843				
119.	*Portulaca quadrifida* L. MUH-1844	Jungle kulfa	Protulacaceae	Whole plant	Extract of whole plant is used treat different diseases like antibacterial, anti-inflammatory
120.	*Phyllanthus niruri* L.	Gale of the wind	Phyllanthaceae	Whole plant	Used to cure liver diseases in the form of powder three times daily, anti-inflammatory, antibacterial, antiseptic, liver diseases, diuretic.
	MUH-1845				
121.	*Polygonum plebeium* L. MUH-1846	Knotweed	Polygonaceae	Whole plant	Extract of plant is used to cure different diseases like tonic, treat pneumonia, fever
122.	*Polygonum aviculare* L. MUH-1847	Weed	Polygonaceae	Rhizome	Rhizome infusion is used for the treatment of diseases like against cough, dysentery, diarrhea.
123.	*Polygonatum multiflora* L.	Soolmoon seal	Polygonaceae	Rhizome	Make a paste of rhizome of plant and used to cure different diseases like dysentery, fever, antiseptic, antibacterial, diarrhea.
	MUH-1848				
124.	*Portulaca oleracea* L.	Zangali Warkhrhay	Portulacaceae	Whole plant	Taken leaves cocked as food and used treatment of different diseases. Leaves also used to cure skin diseases externally.
	MUH-1849				
125.	*Rumex acetosella* L.	Garden sorrel	Polygonaceae	Stem, leaves	Decoction of aerial parts of plant used to cure different diseases like jaundice, urinary, antiseptic, diuretic
	MUH-1854				
126.	*Rumex dentatus* L.	Toothed duck	Polygonaceae	Root and leaves	Root and leaves extract are used to cure skin diseases like wound healing, coetaneous disorder.
	MUH-1855				
127.	*Rumex obtusifolius* L.	Jungle palak	Polygonaceae	Whole plant	Infusions of different plants are used to treat different diseases like kidney diseases, colds, cough, asthma
	MUH-1856				
128.	*Rumex chalepensis* Mill. MUH-1857	Hula	Polygonaceae	Whole plant	Extract of whole plant is used to treat different diseases like diuretic, antiseptic, asthma, colds
129.	*Rumex nepalensis* L.	Dock	Polygonaceae	Leaves	Infusion of leaves is used treat different diseases like stomach diseases, tonic, diarrhea
	MUH-1858				
130.	*Ranunculus sceleratus* Linn. MUH-1859	Gul-eashrafi	Ranunculaceae	Leaves, fruit	Extract of leaves is effective for asthma and cure tumors and boils.
131.	*Ranunculus muricatus* L. MUH-1860	Kar-	Ranunculaceae	Whole plant	Plant extract is used to cure different diseases like cough, asthma, snake bite, tumor
		kandoli			
132.	*Ranunculus arvensis* L. MUH-1861	Corn buttercup	Ranunculaceae	Whole plant	Paste of whole plant is used treat different diseases like wound healing, skin diseases
133.	*Ranunculus laetus* L. MUH-1862	Chambal booti	Ranunculaceae	Leaves	Paste of fresh leaves applied on wounds
134.	*Solanum surattense* Burm.	Marhaghonay	Solanaceae	Whole plant	Whole plant extract is effective for stomach diseases, cough and fever, chest pain
	MUH-1867				
135.	*Setaria pallidefusca* C.E. Hubb.	Bihari grass	Poaceae	Seeds	Take seed, grind make flour and used to treat skin diseases.
	MUH-1868				
136.	*Saccharum spontaneum* L.	Kaai	Poaceae	Leaves	Ach of whole plant mixed with water and used treat different diseases like blood disorders, constipation, liver diseases.
	MUH-1869				
137.	*Setaria glauca* L.	Green foxtail	Poaceae	Whole plant	Flour of plant is used to treat skin diseases, such as chicken pox.
	MUH-1870				
138.	*Sporobolus helvolus* L. MUH-1871	Smut grass	Poaceae	Whole plant	Whole plant is used as fodder
139.	*Silybum marianum* Gaertn.	Kanndyara	Asteraceae	Whole plant	Whole plant extract is used treat different disease, antidiabetic, treat skin diseases, anticancer, tumor,
	MUH-1872				
140.	*Sonchus arvensis* L.	Sowthistle	Asteraceae	Leaves, root	The extract of leaves is used to treat cough, asthma and cold. The tea of root is used to treat chest pain and anti-inflammatory
	MUH-1873				
141.	*Sonchus asper* (L.) Hell	spiny Sowthistle	Asteraceae	Whole plant	For enhancing milk, shoots give to domestic animals
	MUH-1874				
142.	*Saussurea costus* L.	Kuth	Asteraceae	Root	Root extract is effective for skin disease
	MUH-1875				
143.	*Solanum nigrum* L.	Katch match	Solanaceae	Leaves	Leaves are crushed in green condition and used to cure warts on skin.
	MUH-1876				
144.	*Sisymbrium irio* L.	Weed	Brassicaceae	Whole plant	Whole plant dried, crushed, makes powder and used to cure heart diseases.
	MUH-1877				
145.	*Silene conoidea* L.	Pataki	Caryophyllaceae	Root	Root tract is used as wound healing and juice is used to cure skin diseases, wound healing, malarial fever, stomach diseases, headache
	MUH-1878				
146.	*Sophora mollis* L.	Phagan booti	Fabaceae	Leaves, seed	Powder obtained from seeds is used to cure different diseases including joint diseases, kidney diseases
	MUH-1879				
147.	*Trianthema portulacastrum*	Itsit	Aizoaceae	Whole plant	Powder of whole plant is used to treat different blood related diseases diuretic, night blindness, anticancer.
	L. MUH-1880				
148.	*Thalictrum minus* L.	Meadow-rue	Ranunculaceae	Root	Root extract is very effective for different diseases like diuretic, stomach diseases, fever, skin diseases.
	MUH-1881				
149.	*Themeda antheria* News. MUH-1882	Red grass	Poaceae	Whole plant	Powder of whole plant parts is ground and used to treat wounds.
150.	*Tribulus terrestris* L. MUH-1883	Bullhead	Zygophyllaceae	Whole plant	Whole plant extraction is used to treat different diseases like kidney diseases, diuretic, tonic, stomach diseases.
151.	*Trichodesma indicum* L. MUH-1884	Borage	Boraginaceae	Leaves	Leaf paste is applied on wounds for healing
152.	*Tridax procumbens* L. MUH-1885	Kuthi	Asteraceae	Whole plant	The juice extracted from the leaves is directly applied on wounds, antifungal
153	*Trifolium repens* L.	White clover	Papilionaceae	Whole plant	Plant infusion is used to treat fever. Root extract is used to cure fever and cough.
	MUH-1886				
154.	*Trifolium dubium* L.	Suckling clover	Papilionaceae	Whole plant	Plant extract with water used to cure fever and cold, constipation, antidiabetic, cancer, arthritis
	MUH-1887				
155.	*Trifolium resupinatum* Linn. MUH-1888	Loosin	Papilionaceae	Whole plant	Fodder for animals
156.	*Trichosanthes anguina* L.	Parul	Cucurbitaceae	Leaves	Extract of fresh leaves is used to treat skin diseases, diabetes and ulcer, antimicrobial, antidiabetic, diuretic, cure ulcers
	MUH-1889				
157.	*Thymus serpyllum* L.	Wild thyme	Lamiaceae	Shoot	Take shoot of plant make tea with water and used to cure different diseases like fever, constipation, body pain
	MUH-1890				
158.	*Taraxacum officinale* L. MUH-1891	Hand	Asteraceae	Leaves	Leaves boiled, make paste with salt and haldi used to cure bones
159.	*Typha elephantina* Pers. MUH-1894	Koondar	Typhaceae	Leaves and rhizome	Extract of fresh leaves are used to treat stomach related diseases, dysentery
160.	*Vaccaria hispanica* (Mill.) Rauschert MUH-1899	Masna	Caryophyllaceae	seeds,	A decoction is used to treat different diseases, menstrual problem, skin problems, breast tumor
161.	*Viola canescens* Wall.ex Roxb.	Banafsha	Violaceae	Flowers	Take flowers mixed with sugar make kahwa to treat cough, fever, sore throat.
	MUH-1900				
162.	*Vicia sativa* Retz.	-	Papilionaceae	Whole plant	Plant is dried make powder used with water to cure diseases, cure asthma, cough, skin diseases, tonic, diuretic
	MUH-1901				
163.	*Vallaris solanacea* (Roth) O. Kuntze. MUH-1902	Dhudi	Apocynaceae	Whole plant	Paste of whole plant is used to treat different diseases like antimicrobial, antidiabetic, skin infection, wound healing.
164.	*Veronica anagallis* L. MUH-903	Hazar booti	Scrophulariaceae	Whole plant	Medicines are used to treat throat diseases.
165.	*Veronica thapsus* L.	-	Scrophulariaceae	Leaves	Leaves of plant are used to treat different diseases like tonic other skin diseases
	MUH-1904				
166.	*Veronica polita* Fr.	Sriri	Plantaginaceae	Plant juice	Juice or extract of plant is used treat cuts, burns, sore throat infection
	MUH-1905				
167.	*Vicia sativa* L.	_	Papilionaceae	Whole plant	Powder of whole plant is used to treat different diseases like antimicrobial, antioxidant, antidiabetic, diuretic.
	MUH-1906				
168.	*Vicia hirsuta* L.	-	Papilionaceae	Whole plant	Powder of whole plant is used to treat different diseases like diuretic, antidiabetic, antioxidant, antimicrobial
	MUH-1907				
169.	*Vicoa indica* L. MUH-1908	Golden daisy	Asteraceae	Whole plant	Leaves are boiled with water and used orally to treat different diseases like dysentery and other digestive diseases
170.	*Valeriana wallichii*	Mushkbala	Valerianaceae	Whole plant	Powder of whole plant is used to treat different diseases like sedative, stomachic, obesity, snake poisoning, nervous disorders and skin diseases.
	L. MUH-1909				
171.	*Withania somnifera* L.	Dodak	Solanaceae	Root, fruit	Make powder of root or fruit and used with milk or honey to cure nervous disorders, ulcers, anti-inflammatory
	MUH-1910				
172.	*Woodfordia fruticosa*	Tahvi	Lythraceae	Whole plant	Powder of whole plant is used to treat different diseases like fever, dysentery, toothache
	(L.) Kurz				
	MUH-1911				
173.	*Xanthium strumarium* L. MUH-1912	Bakhra	Asteraceae	Whole plant	Leaves are crushed and used for curing different diseases like small pox, malarial fever, dysentery and poisons.

Different parts of plants used for the treatment of different disease. Plant leaves are used up to 62.8%, 8.5% whole plant, 28.0% fruit, 11.4% roots of plants and 8.5% flowers, 8.5% seeds, 28.5% resins or gums and 20.0% stem were used to treat different diseases. (Table 5, Fig 3). The similar results have been reported in earlier works that had been directed in Island and Italy which described that the leaves were frequently used in herbal medicines [39, 40]. It has been found that extreme assembly of leaves along with other plant parts like bark and roots because leaves have more efficiency than other parts because leaf has a greater number of chemical ingredients [41].

**Fig 3:** %age of plant parts used to treat different diseases of SMR of District Bhimber of AJK, Pakistan.

**Table 5:** %age of plant parts used to treat different diseases of SMR of District Bhimber of AJK, Pakistan.

S. No.	Plant parts	%age	S. No.	Plant parts	%age
01	Whole plant	45.0	05	Seeds	10.4
02	Leaves	28.3	06	Fruits	3.4
03	Stem	1.60	07	Flowers	5.2
04	Root	9.2			

### Informant Consensus Factor (ICF) and Fidelity Level (FL)

The major aliments were classified into 12 disease categories by using ICF. According to ICF values the highest numbers of plant species were used against wound healing, snake bite, skin diseases, eye diseases and asthma (Table 6; Fig 4). *Brassica campestris* L. with maximum FL (40.0) followed by *Aloe vera* L. with FL (36.6%) and *Adiantum capillus-veneris* L. with FL (30.0%) were used as antidiabetic and skin diseases, arthritis, respectively (Table 7). Similar findings were also conducted by Ishtiaq *et al*., 2021 [3]. ICF results for ethnomedicines were fluke with past investigators available by different experts in respite of the world [42]. The ICF values of the diseases occurring in the area were similar with past studies conducted in different areas of Pakistan [43] and Azad Kashmir [36, 44].

**Fig 4:** ROP value of indigenous plants species from SMR District Bhimber of AJK, Pakistan.

**Table 6:** Informant Consensus Factor (ICF) of herbal flora of SMR area of District Bhimber, AJK.

Pakistan					
S. No.	Categories	No. of species(nt)	%age of species	No. of Use citation (nur)	$ICF=\frac{nur-nt}{nur-1}$
01	Skin diseases	04	21.9	11	0.7
02	Wound healing	08	16.7	18	1.1
03	Fever	09	14.4	24	0.6
04	Stomach diseases	09	17.3	12	0.3
05	Cough curing	06	12.13	14	0.6
06	Cancer	04	22.7	17	0.9
07	Jaundice	06	17.14	13	0.5
08	Asthma	03	4.6	11	0.8
09	Tooth problems	07	1.7	10	0.3
10	Kidney diseases	06	8.09	13	0.6
11	Diabetes	04	9.2	17	0.8
12	Snake biting	03	4.62	19	0.9

**Table 7:** Fidelity Level (FL), RPL and ROP of some dominant herb species used to treat some diseases in study area (total number of informants = 35).

Botanical name of plants	Major aliment	Np	FL = Np /N×100	RPL	ROP = FL×RPL
*Achyranthes aspera* L.	Constipation	04	13.3%	0.4	5.32
*Amaranthus viridis* L.	Wound healing	02	6.66%	0.2	1.33
*Alternanthera pungens* L.	Anticancer	05	16.6%	0.8	1.32
*Anagallis arvensis* L.	Stomach diseases	03	10.0%	1.0	10.0
*Artemisia maritime* L.	Constipation	01	3.33%	0.6	1.99
*Achillea millefolium* L.	Wound healing	03	10.0%	0.3	3.00
*Aloe vera* L.	Skin diseases, arthritis	11	36.6%	0.9	3.29
*Adiantum capillus-veneris* L.	Hypertension	09	30.0%	0.3	0.90
*Boerhavia diffusa* L.	Kidney diseases	04	13.3%	0.5	6.65
*Brassica campestris* L.	Antidiabetic	12	40.0%	0.1	4.00
*Bryophyllum pinnatum* L.	Wound healing	01	3.33%	1.0	0.33
*Carthamus oxycantha* L.	Skin diseases	04	13.3%	0.4	0.54
*Chenopodium album* L.	Kidney disorders	08	26.6%	0.8	2.12
*Convolvulus arvensis* L.	Constipation	01	3.33%	0.4	0.13
*Cuscuta reflexa* Roxb.	Skin diseases	01	3.33%	0.9	0.29
*Cynodon dactyolon* L.	Wound healing	03	10.0%	0.1	1.00
*Cordia obliqua* L.	Ulcers	04	13.3%	0.5	0.66
*Cyperus esculentus* L.	Antidiabetic	02	6.66%	0.4	0.26
*Cyperus rotundus* L.	Digestive diseases	05	16.6%	0.7	11.6
*Citrullus lanatus* L.	Anticancer	03	10.0%	0.3	3.00
*Citrullus colocynthis* L.	Ulcers	02	6.66%	1.0	6.66
*Coronopus didymus* L.	Inflammatory	01	3.33%	0.5	1.66
*Carssia opaca* L.	Wound healing	01	3.33%	0.9	0.29
*Dicliptera roxburghiana* Nees.	Skin diseases	05	16.6%	0.6	9.96
*Dichanthium annulatum* Forssk.	Dysentery	02	6.66%	0.9	5.99
*Euphorbia hirta* L.	Diarrhea	04	13.3%	0.3	3.99
*Euphorbia helioscopia* L.	Skin diseseaes	02	6.66%	0.5	3.33
*Eclipta prostrate* L.	Kidney diseases	02	6.66%	0.6	3.99
*Ficus auriculata* L.	Diarrhea	01	3.33%	0.7	2.33
*Fumaria indica* L.	Digestive diseases	03	10.0%	0.2	2.00
*Ficus variegata* L.	Constipation	01	3.33%	1.0	3.33
*Gallium elegans* L.	Constipation	03	10.0%	0.7	7.00
*Heteropogon contortus* L.	Wound healing	01	3.33%	0.9	2.99
*Hordeum vulgare* L	Cure jaundice	07	23.3%	0.4	9.32
*Imperata cylindrica* L.	Dysentery	03	10.0%	0.3	3.00
*Lythrus aphaca* L.	Anti-inflammatory	01	3.33%	0.7	2.33
*Leucas aspera* L.	Cough curing	02	6.66%	0.4	2.66
*Malva parviflora* L.	Ulcers	05	16.6%	0.8	13.3
*Melilotus alba* L.	Dysentery	01	3.33%	0.9	2.99
*Mentha royleana* Benth.	Throat pain	01	3.33%	0.4	1.32
*Oxalis corniculata* L.	Skin diseases	01	3.33%	0.1	0.33
*Ocimum bacilicum* L.	Cure cough	01	3.33%	1.0	3.33
*Ocimum sanctum* L.	Heart diseases	04	13.3%	1.0	13.3
*Opuntia dillenii* Haw.	Ulcer	01	3.33%	0.2	0.66
*Parthenium hysterophorus* L.	Antidiabetic	02	6.66%	0.7	4.66
*Papaver dubium* L.	Cough curing	01	3.33%	0.9	2.99
*Phalaris minor* L.	Dysentery	04	13.3%	0.5	6.65
*Portulaca quadrifida* L.	Antibacterial	03	10.0%	0.6	6.00
*Rumex dentatus* L.	Skin diseases	01	3.33%	0.2	0.66
*Rumex obtusifolia* L.	Kidney diseases	05	16.6%	0.8	13.3
*Ranunculus sceleratus* L.	Asthma	03	10.0%	0.5	5.00
*Ranunculus laetus* L.	Skin diseases	06	20.0%	0.9	18.0
*Saccharum spontaneum* L.	Constipation	01	3.33%	0.3	0.99
*Silybum marianum* Gaerth.	Antidiabetic	01	3.33%	0.6	1.99
*Solanum nigrum* L.	Stomach diseases	06	20.0%	0.7	14.0
*Silene conoidea* L.	Malarial fever	05	16.6%	0.4	6.64
*Taraxacum officinales* L.	Arthritis	02	6.66%	0.1	0.66
*Viola canescens* L.	Cough curing	02	6.66%	0.7	4.66
*Withania somnifera* L.	Ulcers	03	10.0%	1.0	10.0
*Withania coagulants* L.	Arthritis	01	3.33%	0.6	1.99
*Xanthium stramonium* L.	Malarial fever	02	6.66%	0.8	5.32
*Youngia japonica* L.	Wound healing	01	3.33%	0.3	0.99

## Relative Frequency Citation (RFC) and Use Value (UV) of ethnobotanical uses of herbs

Ethnobotanical significance of many herbs was calculated by using relative frequency of citation (RFC) and use value (UV). These quantitative values shown the trend of ethnobotanically used plants in respected area. The UV of different herb species was ranges within 0.29 to 0.57. Highest value was calculated for *Alternanthera pungens* L. (0.57), then for *Achyranthes aspera* L. (0.44), while lowest was recorded for *Adiantum capillus-veneris* L. (0.29). RFC value was calculated on the bases of the response of the interviewers recorded during survey section. Highest relative frequency was measured for *Alternanthera pungens* L. (RFC = 51) and lowest was measured for *Adiantum capillus-veneris* L. (RFC = 20). RFC values represent the relative popularity of individual species in study area according to their use. RFC and UV of common plants are listed in (Table 8). Similar findings were reported by the previous researchers who depicted that quantitative tools are very valuable in analysis of significance of each species. Coinciding results were provided in the past works who stated that these cited species of high medicinal value and can be used for drug discovery through analytical studies [45, 46].

**Table 8:** Relative Frequency of Citation (RFC) and Use Value (UV) and of different important EB plants from SMR District Bhimber AJK, Pakistan.

Sr. No.	Names of plants	Common name	Family	Ethnobotanical Use	RFC	UV
01.	*Achyranthes aspera* L. MUH-1681	Phothkanda	Amaranthaceae	Fruit	41	0.44
02	*Astragalus leucocephalus* Benth. MUH-1678	Kathi	Fabaceae	Leaves	38	0.42
03.	*Amaranthus viridis* L. MUH-1682	Ganar	Amaranthaceae	Whole plant	33	0.33
04.	*Amaranthus tricolor* L. MUH-1683	Bhaji	Amaranthaceae	Leaves, root	28	0.31
05.	*Achyranthes bidentata* L. MUH-1684	Phothkanda	Amaranthaceae	Whole plant	43	0.43
06.	*Aerva javanica* (Burm.f.) Juss. MUH-1685	Bui	Amaranthaceae	Whole plant	27	0.36
07.	*Anagallis arvensis* L. MUH-1686	Bili booti	Primulaceae	Leaves	33	0.38
08.	*Abutilon indicum* L. MUH-1687	Sweet kangi	Malvaceae	Whole plant	38	0.33
09.	*Aerva sanguinolenta* (L.)Blume. MUST-1688	Chiti boti	Amaranthaceae	Whole plant	49	0.43
10.	*Alternanthera pungens* L. MUH-1689	Taahee booti	Amaranthaceae	Whole plant	51	0.57
11.	*Argemone mexicana* L. MUH-1690	Dudhli kandyari	Papaveraceae	Whole plant	31	0.41
12.	*Artemisia scoparia* Waldst. & Kit. MUH-1691	Red stem	Asteraceae	Leaves, flowers	27	0.43
13.	*Allium Jacquemontii* Knuth. MUH-1692	Jangli piaz	Alliaceae	Blub, leaves	38	0.36
14.	*Aloe vera* L. MUH-1693	Kawar gandal	Liliaceae	Leaves	31	0.32
15.	*Avena fatua* L. MUH-1695	Wild oat	Poaceae	Seeds	33	0.30
16.	*Acrachne racemosa* L. MUH-1696	Goose grass	Poaceae	Whole plant	38	0.42
17.	*Aristolochia punjabensis* Lace. MUH-1697	Pipevine	Aristolochiaceae	Roots	25	0.41
18.	*Adiantum capillus* L. MUH-1698	Median hair fern	Adiantaceae	Whole plant	20	0.29
19.	*Adiantum incisum* L. MUH-1699	Fern	Adiantaceae	Leaves	38	0.38
20.	*Asplenium trichomanes* L. MUH-1700	Bird nest fern	Caesalpiniaceae	Leaves	27	0.43
21.	*Asphodelus tenuifolius* Caven. MUH-1701	Bhokal	Liliaceae	Seeds	29	0.41
22.	*Ajuga bracteosa* Benth. MUH-1702	Hari booti	Lamiaceae	Whole plant	38	0.38
23.	*Aristida adscensionsis* L. MUH-1703	Saroot	Poaceae	whole plant	28	0.42
24.	*Berberis lyceum* L. MUH-1708	Sumblu	Berberidaceae	Bark	27	0.33
25.	*Boerhavia diffusa* L. MUH-1709	Sanati	Nyctaginaceae	Roots, leaves	40	0.31
26.	*Buglossoides arvensis* L. MUH-1711	Kalu	Boraginaceae	Leaves	33	0.41
27.	*Barleria cristata* L. MUH-1712	-	Acanthaceae	Root, leaves, seeds	36	0.36
28.	*Bryophyllum pinnatum* L. MUH-1713	Pather chatt	Crassulaceae	Leaves	39	0.38
29.	*Bromus japonicus* L. MUH-1714	Broom grass	Poaceae	Whole plant	43	0.33
30.	*Cannabis sativa* L. MUH-1719	Bhang	Cannabaceae	Leaves	49	0.43
31.	*Capparis sepiaria* L. MUH-1720	Kareer	Cyperaceae	Whole plant	33	0.36
32.	*Calendula arvensis* L. MUH-1721	Field marigold	Asteraceae	Leaves and flowers	44	0.41
33.	*Carthamus lanatus* L. MUH-1722	Distaff thistle	Asteraceae	Flowers, seeds	33	0.43
34.	*Calendula officinalis* L. MUH-1723	Marigold	Asteraceae	Leaves, flowers	49	0.36
35.	*Carthamus oxyacantha* L.MUH-1724	Kandyari	Asteraceae	Flowers, seeds	28	0.32
36.	*Chenopodium ambrosioides* L. MUH-1725	Mexicana tea	Chenopodiaceae	Leaves, flowers, and seeds.	21	0.30
37.	*Chenopodium botrys* L. MUH-1726	Oak	Chenopodiaceae	Leaves and seeds	29	0.42
38.	*Chenopodium album* L. MUH-1727	Bathu	Chenopodiaceae	Leaves	25	0.41
39.	*Colebrookea Oppositifolia* Smith. MUH-1728	Bansa	Labiatae	Leaf, root, bark	21	0.33
40.	*Ceropegia bulbosa* L. MUH-1729	Galot	Asclepiadaceae	Tuber, leaves	28	0.38
41.	*Convolvulus arvensis* L. MUH-1730	Rawari	Convolvulaceae	Whole plant	24	0.43
42.	*Cichorium intybus* L. MUH-1731	Kasni	Asteraceae	Seeds, leaves	43	0.41
43.	*Chenopodium ambrosioides* L. MUH-1732	Gandi booti	Chenopodiaceae	Leaf, root	42	0.37
44.	*Cuscuta reflexa* Roxb. MUH-1733	Neel dhari	Cuscutaceae	Whole plant	47	0.42
45.	*Cynodon dactyolon* L. MUH-1734	Khabal	Poaceae	Whole plant	38	0.33
46.	*Cenchrus ciliaris* L. MUH-1735	Ghass	Poaceae	Whole plant	27	0.31
47.	*Cynoglossum lanceolatum* Forrsk. MUH-1736	Leendra	Boraginaceae	Whole plant	21	0.37
48.	*Cordia obliqua* L. MUH-1737	Lasoora	Boraginaceae	Whole plant	28	0.43
49.	*Cassia obtusifolia* L. MUH-1738	Coffee weed	Fabaceae	Leaves, root, seed, flowers	21	0.38
50.	*Cenchrus biflorus* Del MUH-1739	Gass	Poaceae	Leaves and seed	39	0.33
51.	*Cortusa brotheri* L. MUH-1741	-	Primulaceae	Seed and stem	43	0.42
52.	*Cyperus esculentus* L. MUH-1742	Nut sadge	Cyperaceae	Whole plant	49	0.33
53.	*Cyperus iria* L. MUH-1743	Flat sadge	Cyperaceae	Root and fruit	47	0.41
54.	*Cyperus rotundus* L. MUH-1744	Purple sadge	Cyperaceae	Root tubers	42	0.43
55.	*Clitoria ternatea* L. MUH-1745	Butterfly pea	Fabaceae	Stem, flower, leaf, fruit	38	0.36
56.	*Citrullus lanatus* L. MUH-1746	Cheebar	Cucurbitaceae	Seed, leaves	31	0.32
57.	*Citrullus colocynthis* L. MUH-1747	Tumma	Cucurbitaceae	Root and fruit	28	0.30
58.	*Coronopus didymus* L. MUH-1749	Jangliu halon	Brassicaceae	Whole plant	23	0.32
59.	*Carissa opaca* L.MUH-1750	Amaltas	Caesalpiniaceae	Root	43	0.41
60.	*Digera muricata* L. MUH-1752	-	Poaceae	Whole plant	39	0.33
61.	*Dicliptera roxburghiana* News. MUH-1755	Kali boti	Acanthaceae	Plant sap, leaves, flower	42	0.38
62.	*Dicliptera bupleuroides* News. MUH-1756	Marvel grass	Poaceae	Whole plant	38	0.43
63.	*Dichanthium annulatum* Forssk. MUH-1757	Crabgrass	Poaceae	Whole plants	33	0.41
64.	*Digitaria ciliaris* Retz. MUH-1758	Finger grass	Poaceae	whole plant	25	0.34
65.	*Digitaria nodosa* L. MUH-1759	Grass crow foot	Poaceae	whole plant	26	0.42
66.	*Equisetum arvensis* L. MUH-1764	Horsetail	Equisetaceae	Whole plant	29	0.33
67.	*Euphorbia hirta* L. MUH-1765	Dhodke	Euphorbiaceae	Seeds	31	0.31
68	*Euphorbias prostate* L. MUH-1766	Sand mat	Euphorbiaceae	Whole plant	28	0.33
69.	*Euphorbia helioscopia* L. MUH-1767	Cathri dodak	Euphorbiaceae	Whole plant	31	0.36
70.	*Euphorbia prolifera* L. MUH-1768	Dodak	Euphorbiaceae	Whole plant	49	0.38
71.	*Eclipta prostrata* L. MUH-1769	Flase daisy	Asteraceae	Whole plant	42	0.33
72.	*Evolvulus alsinoides* L. Bioss. MUH-1770	Morning glory	Poaceae	Leaves	43	0.31
73	*Echinochloa crus-galli* L. MUH-1771	Cockspur grass	Poaceae	Shoots, roots, seed	44	0.35
74.	*Eleusine indica* L. MUH-1772	Goose grass	Poaceae	Whole plant	47	0.41
75.	*Ehretia laevis* Roxb. MUH-1773	Sakkar	Boraginaceae	Whole plant	41	0.43
76.	*Fumaria indica* L. MUH-1780	Papra	Fumariaceae	Whole plant	43	0.36
77.	*Galium aparine* L. MUH-1784	Lahndara	Rubiaceae	Whole plant	39	0.32
78	*Galium elegans* L. MUH-1785	Jari	Rubiaceae	Whole plant	29	0.30
79.	*Gagea elegans* Wall. MUH-1786	Yellow star	Liliaceae		31	0.43
80.	*Heteropogon contortus* L.MUH-1788	Sarala grass	Poaceae	Whole plant	29	0.39
81.	*Heliotropium strigosu*m Willd. MUH-1789	Gorakh pan	Boraginaceae	Leaves, stem, root	30	0.33
82.	*Helianthus tuberosus* L. MUH-1790	Artichoke	Asteraceae	Whole plant	28	0.38
83.	*Hyoscyamus niger* L. MUH-1791	Khoob kalan	Solanaceae	Whole plant	32	0.43
84.	*Imperata cylindrica* L. MUH-1793	Grass	Poaceae	Root, flower	30	0.41
85.	*Ipomoea eriocarpa* R.Br. MUH-1794	Wanweer booti	Convolvulaceae	Whole plant	28	0.37
86.	*Kyllinga brevifolia* Rottb. MUH-1799	-	Cyperaceae	Rhizome, leaves, tubers	34	0.42
87.	*Loranthus longiflorus* Desr. MUH-1800	Purakh	Loranthaceae	Flowers, leaves	40	0.33
88	*Lantana camara* L. MUH-1801	Panj pholi	Verbenaceae	Leaves	38	0.31
89.	*Larotalaria medicaginea* Lam. MUH-1, 803	Rattle pods	Fabaceae	Whole plant, leaves	31	0.33
90.	*Lathyrus aphaca* L. MUH-1804	jangle matr	Fabaceae	Whole plant	43	0.36
91	*Leucas aspera* L. MUH-1805	Thumbai	Labiatae	Whole plant	28	0.38
92.	*Launaea procumbens* Roxb.MUH-1806	Bathala	Asteraceae	Whole plant	30	0.33
93.	*Maytenus royleana* Wall.MUH-1811	Patakee	Celastraceae	Bark, leaves	43	0.41
94.	*Malva parviflora* L. MUH-1812	Sonchal	Malvaceae	Whole plant	39	0.42
95.	*Malva sylvestris* L. MUH-1813	High mallow	Malvaceae	Seeds	48	0.41
96.	*Melilotus alba* L. MUH-1814	Shinji	Fabaceae	Leaves	41	0.33
97.	*Micromeria biflora* L. MUH-1815	Marathi	Leguminosae	Leaves, root	35	0.36
98.	*Melilotus indica* (L.) All.MUH-1816	jangle methi	Papilionaceae	Leaves	27	0.32
99.	*Medicago polymorpha* L. MUH-1817	Sriri	Papilionaceae	Whole plant	29	0.30
100.	*Mentha royleana* Benth. MUH-1818	Wild mint	Labiatae	Leaves, stem	31	0.42
101.	*Nasturtium officinale* R.Br. MUH-1820	Chooch	Brassicaceae	Leaves	39	0.41
102.	*Nicotiana plumbaginifolia* Viv. MUH-1821	Jangli tobacco	Solanaceae	Whole plant	41	0.33
103.	*Otostegia limbata* L. MUH-1822	Kori booti	Lamiaceae	Leaves	38	0.38
104.	*Oxalis corniculata* L. MUH-1823	Khati boti	Oxalidaceae	Fruits and seeds	39	0.43
105.	*Ocimum bacilicum* L. MUH-1824	Naiazbu	Lamiaceae	Leaves, seeds	28	0.41
106.	*Ocimum tenuiflorum* L. MUH-1825	Tulsi	Lamiaceae	Leaves	30	0.33
107.	*Opuntia dillenii* Haw. MUH-1826	Thor	Cactaceae	Stem	27	0.42
108.	*Polygonum plebeium* L. MUH-1829	-	Polygonaceae	Whole plant	43	0.33
109.	*Persicaria barbata* L. MUH-1830	Jor booti	Polygonaceae	Whole plant	38	0.31
110.	*Parthenium hysterophorus* L. MUH-1835	-	Asteraceae	Whole plant	49	0.41
111.	*Plantago lanceolata* L. MUH-1836	-	Plantaginaceae	Leaves	41	0.36
112.	*Prosopis farcta* L.C. VC. HB. MUH-1837	-	Plantaginaceae	Bark, flowers	31	0.38
113.	*Papaver dubium* L. MUH-1838	Jungle post	Papaveraceae	Flowers, stem	27	0.33
114.	*Panicum turgidum* ForsskMUH-1839	-	Poaceae	Whole plant	38	0.41
115.	*Pennisetum flaccidum* Griseb. MUH-1840	Fountain grass	Poaceae	Whole plant	31	0.34
116.	*Phragmitis karka* (Retz.) MUH-1841	Babyoon	Poaceae	Whole plant	44	0.41
117.	*Poa annua* L. MUH-1842	Grass	Poaceae	Leaves	38	0.43
118.	*Phalaris minor* L. MUH-1843	Bunch grass	Poaceae	Leaves, fruit, seed	25	0.36
119.	*Portulaca quadrifida* L. MUH-1844	Jungle kulfa	Protulacaceae	Whole plant	32	0.32
120.	*Phyllanthus niruri* L. MUH-1845	Gale of the wind	Phyllanthaceae	Whole plant	38	0.30
121.	*Polygonum plebeium* L. MUH-1846	Knotweed	Polygonaceae	Whole plant	27	0.41
122.	*Polygonum aviculare* L. MUH-1847	Weed	Polygonaceae	Rhizome	29	0.33
123.	*Polygonatum multiflora* L. MUH-1848	Soolmoon seal	Polygonaceae	Rhizome	38	0.38
124.	*Portulaca oleracea* L. MUH-1849	Zangali Warkhrhay	Portulacaceae	Whole plant	28	0.37
125.	*Rumex acetosella* L. MUH-1854	Garden sorrel	Polygonaceae	Stem, leaves	31	0.43
126.	*Rumex dentatus* L. MUH-1855	Toothed duck	Polygonaceae	Root and leaves	40	0.41
127.	*Rumex obtusifolius* L. MUH-1856	Jungle palak	Polygonaceae	Whole plant	33	0.42
128.	*Rumex chalepensis* Mill. MUH-1857	Hula	Polygonaceae	Whole plant	36	0.35
129.	*Rumex nepalensis* L. MUH-1858	Dock	Polygonaceae	Leaves	39	0.33
130.	*Ranunculus sceleratus* Linn. MUH-1859	Gul-eashrafi	Ranunculaceae	Leaves, fruit	43	0.31
131.	*Ranunculus muricatus* L. MUH-1860	Kar-kandoli	Ranunculaceae	Whole plant	49	0.41
132.	*Ranunculus arvensis* L. MUH-1861	Corn buttercup	Ranunculaceae	Whole plant	31	0.36
133.	*Ranunculus laetus* L. MUH-1862	Chambal booti	Ranunculaceae	Leaves	44	0.38
134.	*Solanum surratense* Burm.MUH-1867	Marhaghonay	Solanaceae	Whole plant	37	0.33
135.	*Setaria pallidefusca* C.E. Hubb.MUH-1868	Bihari grass	Poaceae	Seeds	49	0.48
136.	*Saccharum spontaneum* L. MUH-1869	Kaai	Poaceae	Leaves	28	0.41
137.	*Setaria glauca* L. MUH-1870	Green foxtail	Poaceae	Whole plant	21	0.43
138.	*Sporobolus helvolus* L. MUH-1871	Smut grass	Poaceae	Whole plant	29	0.33
139.	*Silybum marianum* Gaertn. MUH-1872	Kanndyara	Asteraceae	Whole plant	25	0.36
140.	*Sonchus arvensis* L. MUH-1873	Sowthistle	Asteraceae	Leaves, root	21	0.32
141.	*Sonchus asper* (L.) Hell MUH-1874	spiny Sowthistle	Asteraceae	Whole plant	28	0.30
142.	*Saussurea costus* L. MUH-1875	Kuth	Asteraceae	Root	24	0.42
143.	*Solanum nigrum* L. MUH-1876	Katch match	Solanaceae	Leaves	33	0.41
144.	*Sisymbrium irio* L. MUH-1877	Weed	Brassicaceae	Whole plant	42	0.32
145.	*Silene conoidea* L. MUH-1878	Pataki	Caryophyllaceae	Root	47	0.38
146.	*Sophora mollis* L. MUH-1879	Phagan booti	Fabaceae	Leaves, seed	38	0.43
147.	*Trianthema portulacastrum* L. MUH-1880	Itsit	Aizoaceae	Whole plant	27	0.41
148.	*Thalictrum minus* L. MUH-1881	Meadow-rue	Ranunculaceae	Root	21	0.43
149.	*Themeda antheria* News. MUH-1882	Red grass	Poaceae	Whole plant	28	0.42
150.	*Tribulus terrestris* L. MUH-1883	Bullhead	Zygophyllaceae	Whole plant	21	0.33
151.	*Trichodesma indicum* L. MUH-1884	Borage	Boraginaceae	Leaves	39	0.31
152.	*Tridax procumbens* L. MUH-1885	Kuthi	Asteraceae	Whole plant	43	0.41
153	*Trifolium repens* L. MUH-1886	White clover	Papilionaceae	Whole plant	49	0.36
154.	*Trifolium dubium* L. MUH-1887	Suckling clover	Papilionaceae	Whole plant	47	0.38
155.	*Trifolium resupinatum* Linn. MUH-1888	Loosin	Papilionaceae	Whole plant	42	0.33
156.	*Trichosanthes anguina* L. MUH-1889	Parul	Cucurbitaceae	Leaves	38	0.40
157.	*Thymus serpyllum* L. MUH-1890	Wild thyme	Lamiaceae	Shoot	31	0.37
158.	*Taraxacum officinale* L. MUH-1891	Hand	Asteraceae	Leaves	28	0.41
159.	*Typha elephantina* Pers. MUH-1894	Koondar	Typhaceae	Leaves and rhizome	23	0.43
160.	*Vaccaria hispanica* (Mill.) Rauschert MUH-1899	Masna	Caryophyllaceae	seeds,	43	0.36
161.	*Viola canescens* Wall.ex Roxb. MUH-1900	Banafsha	Violaceae	Flowers	39	0.32
162.	*Vicia sativa* Retz. MUH-1901	-	Papilionaceae	Whole plant	42	0.30
163.	*Vallaris solanacea* (Roth) O. Kuntze. MUH-1902	Dhudi	Apocynaceae	Whole plant	38	0.42
164.	*Veronica anagallis* L. MUH-903	Hazar booti	Scrophulariaceae	Whole plant	33	0.41
165.	*Veronica thapsus* L. MUH-1904	-	Scrophulariaceae	Leaves	25	0.33
166.	*Veronica polita* Fr. MUH-1905	Sriri	Plantaginaceae	Plant juice	33	0.38
167.	*Vicia sativa* L. MUH-1906	_	Papilionaceae	Whole plant	29	0.43
168.	*Vicia hirsuta* L. MUH-1907	-	Papilionaceae	Whole plant	31	0.41
169.	*Vicoa indica* L. MUH-1908	Golden daisy	Asteraceae	Whole plant	28	0.38
170.	*Valeriana wallichii* L. MUH-1909	Mushkbala	Valerianaceae	Whole plant	31	0.42
171.	*Withania somnifera* L. MUH-1910	Dodak	Solanaceae	Root, fruit	49	0.33
172.	*Woodfordia fruticosa* (L.) Kurz MUH-1911	Tahvi	Lythraceae	Whole plant	42	0.31
173.	*Xanthium strumarium* L. MUH-1912	Bakhra	Asteraceae	Whole plant	43	0.34

## Relative frequency citation RFC and use value UVI of ethnomedicinal uses trees

Ethnobotanical significance of various plants was calculated by using relative frequency of citation (RFC) and use value index (UVI). These quantitative values depicted the trend of ethnobotanically used plants in respected area. Highest value was calculated for *Alternanthera pungens* L. (0.90), then for *Achyranthes aspera* L. (0.80), while lowest was recorded for *Adiantum capillus* L. (0.29). RFC value was calculated on the bases of the response of the interviewers recorded during survey section. Highest relative frequency was measured for *Alternanthera pungens* L. (RFC = 51) and lowest was measured for *Adiantum capillus* L. (RFC = 20). RFC values represent the relative popularity of individual species in study area according to their use. RFC and UVI of common plants are listed in (Table 9). Similar findings have been reported in previous research work, where herbal has been predominantly used as source of medicines and other life sustenance materials [47–49].

**Table 9:** The Use Value Index (UVI) and Relative Frequency of Citation (RFC) of the most commonly used medicinal plants by the local people of different areas of SMR of District Bhimber (AJK), Pakistan.

S No	Names of plants	Common name	Family	Ethnomedicinal uses	RFC	ƩUi	UV	UVi
1.	*Achyranthes aspera* L. MUH-1681	Phothkanda	Amaranthaceae	Fruits are roosted and grinded and used against asthma, fever, cough, constipation	33	28	0.35	0.80
2.	*Astragalus leucocephalus* Benth. MUH-1678	Kathi	Fabaceae	Powder of leaves is used to cure stomach pain, gastrointestinal pain, kidney diseases.	28	21	0.48	0.60
3.	*Amaranthus viridis* L. MUH-1682	Ganar	Amaranthaceae	Plant is taken dried, make powder and used with water to cure control bleeding, diarrhea, wound healing.	27	22	0.41	0.62
4.	*Amaranthus tricolor* L. MUH-1683	Bhaji	Amaranthaceae	Extract of leaves are effective for snake bite, diuretic and wound healing.	23	27	0.36	0.74
5.	*Achyranthes bidentata* L. MUH-1684	Phothkanda	Amaranthaceae	Ethanolic extract of leaves used for healing wounds, diuretic, treat cancer, eye related diseases and anemia.	21	18	0.26	0.51
6.	*Aerva javanica* (Burm.f.) Juss. MUH-1685	Bui	Amaranthaceae	Extract of plant used to cure different diseases like anti-diarrheal, antimicrobial, cure kidney diseases.	30	29	0.45	0.78
7.	*Anagallis arvensis* L. MUH-1686	Bili booti	Primulaceae	Leaf extract is used to treat stomach diseases, antifungal and wound healing	25	31	0.41	0.70
8.	*Abutilon indicum* L. MUH-1687	Sweet kangi	Malvaceae	Paste of seeds and leaves to cure skin diseases. Aerial parts are used to cure asthma, anti-diarrheal, anticancer, anti-inflammatory and antidiabetic	29	30	0.36	0.73
9.	*Aerva sanguinolenta* (L.) Blume. MUST-1688	Chiti boti	Amaranthaceae	Extract of plant used to cure different diseases anti-diarrheal, antimicrobial and cure kidney diseases.	30	23	0.32	0.65
10.	*Alternanthera pungens* L. MUH-1689	Taahee booti	Amaranthaceae	Ethanolic extract of leaves used for healing wounds, diuretic, treat cancer, eye related diseases and anemia.	51	21	0.27	0.90
11.	*Argemone mexicana* L. MUH-1690	Dudhli kandyari	Papaveraceae	Extract of whole plant used to treat different diseases like wound healing, anti-inflammatory, antibacterial, diuretic, anticancer	22	24	0.42	0.68
12.	*Artemisia scoparia* Waldst. & Kit. MUH-1691	Red stem	Asteraceae	Leaves are dried and made paste used with water to cure stomach diseases, intestinal diseases	29	26	0.48	0.74
13.	*Allium Jacquemontii* Knuth. MUH-1692	Jangli piaz	Alliaceae	Juice of plant parts used to treat different disease like snake bite, scorpion bite and antimicrobial	28	29	0.35	0.72
14.	*Aloe vera* L. MUH-1693	Kawar gandal	Liliaceae	Leaf pulp is applied on wounds for healing and pulp is mixed with sugar used against cardiovascular diseases anticancer, anti-diabetes, cardiovascular diseases.	28	21	0.31	0.62
15.	*Avena fatua* L. MUH-1695	Wild oat	Poaceae	Seed’s grind and powder is used for curing diseases to cure skin diseases and cardiovascular diseases	22	27	0.43	0.77
16.	*Acrachne racemosa* L. MUH-1696	Goose grass	Poaceae	fodder for animals	25	29	0.28	0.73
17.	*Aristolochia punjabensis* Lace. MUH-1697	Pipevine	Aristolochiaceae	Powder of root taken with milk to treat body pain and taken with water to cure menstrual problems treat body pain and menstrual problems	31	26	0.36	0.74
18.	*Adiantum capillus* L. MUH-1698	Median hair fern	Adiantaceae	Whole plant is dried, make powder. Small amount of powder is used for lowering blood pressure level, curing cough, fever, hypertension and hair caring.	20	28	0.41	0.50
19.	*Adiantum incisum* L. MUH-1699	Fern	Adiantaceae	Infusion of leaves used for cough and other diseases like fever, body weakness	22	31	0.37	0.73
20.	*Asplenium trichomanes* L. MUH-1700	Bird nest fern	Caesalpiniaceae	Leaf is smoked for chest pain, colds, headache, cure colds and chest pain	28	21	0.31	0.60
21.	*Asphodelus tenuifolius* Caven. MUH-1701	Bhokal	Liliaceae	Seed powder is taken in piles and used to cure other skin diseases.	26	28	0.25	0.70
22.	*Ajuga bracteosa* Benth. MUH-1702	Hari booti	Lamiaceae	Whole plant is effective for diseases. Root powder is used to cure diarrhea. Leaf powder is used to cure malarial fever, cure stomach diseases and dysentery.	22	31	0.37	0.65
23.	*Aristida adscensionsis* L. MUH-1703	Saroot	Poaceae	Fodder for animals	33	28	0.35	0.73
24.	*Berberis lyceum* L. MUH-1708	Sumblu	Berberidaceae	Powder of bark is applied on wounds for healing, Jaundice and tonic.	28	21	0.48	0.60
25.	*Boerhavia diffusa* L. MUH-1709	Sanati	Nyctaginaceae	Roots re crushed boiled in milk used to remove kidney stones. Make leaves powder and used with water to cure different diseases like pneumonia, abscesses.	27	22	0.41	0.62
26.	*Buglossoides arvensis* L. MUH-1711	Kalu	Boraginaceae	Infusion of leaves are sedatives	23	27	0.36	0.74
27.	*Barleria cristata* L. MUH-1712	-	Acanthaceae	Bitter juice used to treat diseases like lung disorders, snake bite, antimicrobial, diabetes and toothache	21	18	0.26	0.51
28.	*Bryophyllum pinnatum* L. MUH-1713	Pather chatt	Crassulaceae	Fresh leaves are warmed and rapped on wound healing	33	28	0.35	0.73
29.	*Bromus japonicus* L. MUH-1714	Broom grass	Poaceae	Powder of whole plant used to treat different disease like chest pain, anti-inflammatory and hepatitis.	28	21	0.48	0.60
30.	*Cannabis sativa* L. MUH-1719	Bhang	Cannabaceae	Make leaves paste used for wound healing. Leaves are narcotics so used to generate pleasant, cure cough, headache, abdominal pain, used for pleasant and excitement.	27	22	0.41	0.62
31.	*Capparis sepiaria* L. MUH-1720	Kareer	Cyperaceae	Decoction of whole plant used to treat disease like antimicrobial, antifungal and skin diseases	23	27	0.36	0.74
32.	*Calendula arvensis* L. MUH-1721	Field marigold	Asteraceae	Extract of leaves are used to cure antiseptic, cure skin diseases and healing of wounds	21	18	0.26	0.61
33.	*Carthamus lanatus* L. MUH-1722	Distaff thistle	Asteraceae	Make paste of seeds and flowers and applied to cure to different skin diseases and fever	33	28	0.35	0.70
34.	*Calendula officinalis* L. MUH-1723	Marigold	Asteraceae	The sap of flowers used to cure skin diseases and treatment of cancer. The external use of plant extract with tincture is effective for wound healing, blood purifier, cure skin disorders, anticancer, anemia and kidney diseases	28	21	0.48	0.60
35.	*Carthamus oxyacantha* L. MUH-1724	Kandyari	Asteraceae	Flowers are used to cure jaundice while oil extract from seeds use to cure skin diseases and cure jaundice	27	22	0.41	0.62
36.	*Chenopodium ambrosioides* L. MUH-1725	Mexicana tea	Chenopodiaceae	Dried leaves are used to treat cancer. Seed oil is used to cure arthritis, skin diseases,	23	27	0.36	0.74
37.	*Chenopodium botrys* L. MUH-1726	Oak	Chenopodiaceae	Fresh leaves extract is used to cure kidney diseases, arthritis, skin diseases, digestive	21	18	0.26	0.64
38.	*Chenopodium album* L. MUH-1727	Bathu	Chenopodiaceae	Leaf juice is used to cure kidney problems and cure spleen	28	21	0.48	0.60
39.	*Colebrookea Oppositifolia* Smith. MUH-1728	Bansa	Labiatae	Powder of plant parts used to treat different diseases like cure flu, fever, wound healing, epilepsy	27	22	0.41	0.62
40.	*Ceropegia bulbosa* L. MUH-1729	Galot	Asclepiadaceae	Juice of plant parts used to treat diseases like anticancer, antimicrobial, kidney disorders, digestive problems	23	27	0.36	0.74
41.	*Convolvulus arvensis* L. MUH-1730	Rawari	Convolvulaceae	Dried powder of plant mixed with gurr to treat constipation. Leaf paste is used to cure skin diseases, cure constipation, anti-inflammation	21	18	0.26	0.61
42.	*Cichorium intybus* L. MUH-1731	Kasni	Asteraceae	Powder of seed used to treat different diseases like fever, kidney problems, vomiting, toothache, blood purifier	33	28	0.35	0.70
43.	*Chenopodium ambrosioides* L. MUH-1732	Gandi booti	Chenopodiaceae	Paste and juice of plant parts used to treat different diseases like wound healing, constipation, skin burns, stomach pains	28	21	0.48	0.60
44.	*Cuscuta reflexa* Roxb. MUH-1733	Neel dhari	Cuscutaceae	Whole plant extract is used to treat viral diseases, juice is used to cure jaundice, warm paste is used to treat headache. Antiviral, treat cough, arthritis, skin disorders and blood purifiers.	28	21	0.48	0.60
45.	*Cynodon dactyolon* L. MUH-1734	Khabal	Poaceae	Paste of fresh plant is applied on wound healing, skin diseases and fever	27	22	0.41	0.62
46.	*Cenchrus ciliaris* L. MUH-1735	Ghass	Poaceae	Plant is crushed and made powder and used for curing different diseases like kidney diseases, tumors, wound healing	23	27	0.36	0.74
47.	*Cynoglossum lanceolatum* Forrsk. MUH-1736	Leendra	Boraginaceae	Bark of plant is used to cure teeth diseases. Root paste is used to cure cough and tuberculosis diseases	21	18	0.26	0.61
48.	*Cordia obliqua* L. MUH-1737	Lasoora	Boraginaceae	Fruit of this herb is used to cure dry cough, fever and chest pain. Bark juice is used to cure tonic diseases. Leaves are also effective for headache and ulcers.	33	28	0.35	0.70
49.	*Cassia obtusifolia* L. MUH-1738	Coffee weed	Fabaceae	Leaves are used to make tea to remove headache. Used to cure vomiting, skin diseases, ulcers, asthma and eye diseases	28	21	0.48	0.60
50.	*Cenchrus biflorus* Del MUH-1739	Gass	Poaceae	Leaf extract is used to treat different diseases, diuretic, digestive, anti-inflammatory, fever, cold	33	28	0.35	0.73
51.	*Cortusa brotheri* L. MUH-1741	-	Primulaceae	Extract of plant used to treat different diseases like stomach pain and constipation	28	21	0.48	0.60
52.	*Cyperus esculentus* L. MUH-1742	Nut sadge	Cyperaceae	Extract of whole plant is used to treat different diseases. Anti-malarial, anti-diarrheal, antidiabetic, antioxidant, antibacterial	27	22	0.41	0.62
53.	*Cyperus iria* L. MUH-1743	Flat sadge	Cyperaceae	Dried parts of plants are used to cure different diseases like cough, chronic, fever, cold, arthritis and cardiac diseases	23	27	0.36	0.74
54.	*Cyperus rotundus* L. MUH-1744	Purple sadge	Cyperaceae	Roots are grinded, make powder and used with water. Cure digestive and uterus pains.	21	18	0.26	0.62
55.	*Clitoria ternatea* L. MUH-1745	Butterfly pea	Fabaceae	Alcohol extract of plant used to treat different diseases like mental illness, antibacterial, antidiabetic, anti-inflammatory.	33	28	0.35	0.71
56.	*Citrullus lanatus* L. MUH-1746	Cheebar	Cucurbitaceae	Dried pulp of leaves and root are used to treat different diseases like constipation, ulcers, cancer	28	21	0.48	0.60
57.	*Citrullus colocynthis* L. MUH-1747	Tumma	Cucurbitaceae	Extract of whole plant is used to treat different diseases like tumor, ulcers, remove pain, swelling	27	22	0.41	0.62
58.	*Coronopus didymus* L. MUH-1749	Jangliu halon	Brassicaceae	Powder of plant is used to treat different diseases like relive pain, inflammatory	23	27	0.36	0.74
59.	*Carissa opaca* L. MUH-1750	Amaltas	Caesalpiniaceae	Powder of dried root is applied on wounds.	21	18	0.26	0.62
60.	*Digera muricata* L. MUH-1752	-	Poaceae	Infusion of plant used to treat stomach diseases, digestive disorders and urinary diseases	23	27	0.36	0.74
61.	*Dicliptera roxburghiana* News. MUH-1755	Kali boti	Acanthaceae	Dried parts of plants are used to treat different diseases like diuretic, skin diseases, toxic	21	18	0.26	0.51
62.	*Dicliptera bupleuroides* News. MUH-1756	Marvel grass	Poaceae	Powder of plant is used treat different diseases like antidiabetic and antimicrobial	21	18	0.26	0.62
63.	*Dichanthium annulatum* Forssk. MUH-1757	Crabgrass	Poaceae	Dried parts of plant are used to treat different diseases like diuretic, tonic, toxic	33	28	0.35	0.73
64.	*Digitaria ciliaris* Retz. MUH-1758	Finger grass	Poaceae	Fodder for animals	28	21	0.48	0.60
65.	*Digitaria nodosa* L. MUH-1759	Grass crow foot	Poaceae	Fodder for animal.	27	22	0.41	0.62
66.	*Equisetum arvensis* L. MUH-1764	Horsetail	Equisetaceae	Plant juice is used for kidney diseases.	23	27	0.36	0.74
67.	*Euphorbia hirta* L. MUH-1765	Dhodke	Euphorbiaceae	Taken seeds make powder seeds are used to cure diarrhea.	21	18	0.26	0.71
68.	*Euphorbias prostate* L. MUH-1766	Sand mat	Euphorbiaceae	Plant is crushed and eats to remove kidney stones.	33	28	0.35	0.74
69.	*Euphorbia helioscopia* L. MUH-1767	Cathri dodak	Euphorbiaceae	Powder of root is used to cure skin diseases.	28	21	0.48	0.60
70.	*Euphorbia prolifera* L. MUH-1768	Dodak	Euphorbiaceae	Whole plant is taken make powder and used to cure diseases.	27	22	0.41	0.62
71.	*Eclipta prostrata* L. MUH-1769	Flase daisy	Asteraceae	Whole plant is taken dried make powder used to cure different diseases like hepatitis, nervous disorders, anemia, skin diseases.	23	27	0.36	0.74
72.	*Evolvulus alsinoides* L. Bioss. MUH-1770	Morning glory	Poaceae	Extract of leaf is taken for constipation, vomiting, indigestion	21	18	0.26	0.71
73.	*Echinochloa crus-galli* L. MUH-1771	Cockspur grass	Poaceae	Seed can be cooked, sieve, bitter flavor used to prevent different diseases like tonic, cure, wound healing, anticancer, antioxidant	33	28	0.35	0.73
74.	*Eleusine indica* L. MUH-1772	Goose grass	Poaceae	Extract of plant parts used to treat different diseases like kidney, diarrhea, eye diseases, dysentery	28	21	0.48	0.60
75.	*Ehretia laevis* Roxb. MUH-1773	Sakkar	Boraginaceae	Extract of different plant parts used to treat diseases, skin cancer, anti-inflammatory, wound healing	27	22	0.41	0.62
76.	*Fumaria indica* L. MUH-1780	Papra	Fumariaceae	Herb is dried make powder and used to treat different diseases like diuretic, cure liver and digestive diseases, cure skin diseases.	23	27	0.36	0.74
77.	*Galium aparine* L. MUH-1784	Lahndara	Rubiaceae	Plant is crushed make powder and used to treatment of different diseases like cure fever, diuretic, wound healing and antiseptic.	21	18	0.26	0.71
78.	*Galium elegans* L. MUH-1785	Jari	Rubiaceae	Taken whole plant dried, crushed and makes powder used with water to cure different diseases like Jaundice, antiseptic, wound healing, fever	29	28	0.41	0.64
79.	*Gagea elegans* Wall. MUH-1786	Yellow star	Liliaceae	Fodder for animals	22	31	0.37	0.71
80.	*Heteropogon contortus* L. MUH-1788	Sarala grass	Poaceae	Powder of plant is used to make medicine against irritability, wound healing, pneumonia, burns, diuretic and obesity	28	21	0.31	0.60
81.	*Heliotropium strigosu*m Willd. MUH-1789	Gorakh pan	Boraginaceae	Gum is used to treat boils. Juice for snake bite, diuretic, sore pain, wound healing and used to treat boils	26	28	0.25	0.72
82.	*Helianthus tuberosus* L. MUH-1790	Artichoke	Asteraceae	Whole pant is used to treat different diseases diuretic, antidiabetics, stomach diseases, tonic effect, antidiabetic, anti-microbial	29	28	0.41	0.74
83.	*Hyoscyamus niger* Linn. MUH-1791	Khoob kalan	Solanaceae	Powder of whole plant is used to treat different diseases like pain killer, kidney stones	22	31	0.37	0.62
84.	*Imperata cylindrica* L. MUH-1793	Grass	Poaceae	A decoction of the root is used to treat digestive diseases, wound healing, antijaundice, dysentery	28	21	0.31	0.60
85.	*Ipomoea eriocarpa* R.Br. MUH-1794	Wanweer booti	Convolvulaceae	Crush whole plant, make powder and extract is used to cure skin diseases, cancer	26	28	0.25	0.71
86.	*Kyllinga brevifolia* Rottb. MUH-1799	-	Cyperaceae	Extract of plant parts used to treat different diseases like digestive, diuretic, tonic, sedative, antimalarial, snake bite	29	28	0.41	0.75
87.	*Loranthus longiflorus* Desr. MUH-1800	Purakh	Loranthaceae	Decoction of plant is used to treat different diseases like diabetes, skin diseases, wound healing, bone repairing	22	31	0.37	0.74
88.	*Lantana camara* L. MUH-1801	Panj pholi	Verbenaceae	Ethanolic extract of leaves are reported for wound healing, Skin diseases, anticancer, anti-inflammatory, malarial diseases.	28	21	0.31	0.60
89.	*Larotalaria medicaginea* Lam. MUH-1, 803	Rattle pods	Fabaceae	Make powder of whole plant and used to treat different diseases like malaria, constipation, fever	26	28	0.25	0.74
90.	*Lathyrus aphaca* L. MUH-1804	jangle matr	Fabaceae	Powder of whole plant is used to treat different diseases like burns, anti-inflammatory, anti-bacterial	33	28	0.35	0.64
91.	*Leucas aspera* L. MUH-1805	Thumbai	Labiatae	Flower are mixed with honey and used for different diseases like fever, cough, cold, ulcer	28	21	0.48	0.60
92.	*Launaea procumbens* Roxb. MUH-1806	Bathala	Asteraceae	Powder of whole plant is used treat different diseases like skin diseases, cough, chest pain, obesity, constipation	27	22	0.41	0.62
93.	*Maytenus royleana* Wall. MUH-1811	Patakee	Celastraceae	Paste of Bark and leaves used for bone fractures and other skin diseases	23	27	0.36	0.74
94.	*Malva parviflora* L. MUH-1812	Sonchal	Malvaceae	Leaves extract with water is used to cure different diseases, anti-inflammatory, antimicrobial	21	18	0.26	0.63
95.	*Malva sylvestris* L. MUH-1813	High mallow	Malvaceae	Seeds are boiled, add sugar made sharabt used to cure fever and cough	26	28	0.25	0.75
96.	*Melilotus alba* L. MUH-1814	Shinji	Fabaceae	Infusion of leaves is used to treat different diseases including dysentery, cough, bronchial disorders, abdominal pain	29	28	0.41	0.72
97.	*Micromeria biflora* L. MUH-1815	Marathi	Leguminosae	Root extract is to cure different diseases. Leaf oil used as flavoring agent, cure dysentery, colds, cough, abdominal pain	22	31	0.37	0.76
98.	*Melilotus indica* (L.) All. MUH-1816	jangle methi	Papilionaceae	Leaf juice is used against antibacterial disorders.	28	21	0.31	0.60
99.	*Medicago polymorpha* L. MUH-1817	Sriri	Papilionaceae	Seed can be ground into a powder and mixed with water and used to treat different diseases like cure skin diseases, dysentery, wound healing	26	28	0.25	0.71
100.	*Mentha royleana* Benth. MUH-1818	Wild mint	Labiatae	Leaves are dried and, make powder used to cure different diseases like cough, throat pain, digestion and constipation.	33	28	0.35	0.0.71
101.	*Nasturtium officinale* R.Br. MUH-1820	Chooch	Brassicaceae	Leaf juice is taken for stomach diseases, ulcers, intestinal pain	28	21	0.48	0.60
102.	*Nicotiana plumbaginifolia* Viv. MUH-1821	Jangli tobacco	Solanaceae	Powder of leaves used to treat different diseases like healing of wounds and cuts toothache, rheumatic	27	22	0.41	0.62
103.	*Otostegia limbata* L. MUH-1822	Kori booti	Lamiaceae	Leaves are dried, grind and powder are applied on wound	23	27	0.36	0.74
104.	*Oxalis corniculata* L. MUH-1823	Khati boti	Oxalidaceae	Plant sap is used to cure skin diseases	21	18	0.26	0.63
105.	*Ocmum bacilicum* L. MUH-1824	Naiazbu	Lamiaceae	Leaf extract is used to cure cough. Seed powder is used in cold drinks.	33	28	0.35	0.72
106.	*Ocimum tenuiflorum* L. MUH-1825	Tulsi	Lamiaceae	Leaves are crushed mixed with water make juice used for treatment of different diseases like cure fever, anticancer, skin disorders, heart related diseases.	28	21	0.48	0.60
107.	*Opuntia dillenii* Haw. MUH-1826	Thor	Cactaceae	Decoction of whole plant is used orally to treat different diseases like asthma, Anti-diabetics, ulcer, Anti-inflammatory, antimicrobial	27	22	0.41	0.62
108.	*Polygonum plebeium* L. MUH-1829	-	Polygonaceae	Extract of plant is used to treat different diseases like pneumonia, liver diseases, heart related disease	23	27	0.36	0.74
109.	*Persicaria barbata* L. MUH-1830	Jor booti	Polygonaceae	Extract of whole plant is used to treat different diseases like kidney stones, ulcers, asthma, sedatives, gastric diseases, insecticides.	21	18	0.26	0.71
110.	*Parthenium hysterophorus* L. MUH-1835	-	Asteraceae	Extract of whole plant is used treat different diseases, anticancer, antidiabetic	33	28	0.35	0.74
111.	*Plantago lanceolata* L. MUH-1836	-	Plantaginaceae	Take leaves of plant make paste and applied on inflamed places.	28	21	0.48	0.60
112.	*Prosopis farcta* L.C. VC. HB. MUH-1837	-	Plantaginaceae	The flowers are mixed with sugar and use to prevent miscarriage. Bark is effective for different diseases like asthma, dysentery, skin diseases, snake bite.	27	22	0.41	0.62
113.	*Papaver dubium* L. MUH-1838	Jungle post	Papaveraceae	Infusion of whole plant is used to treat different diseases like cough, fever, antimicrobial	23	27	0.36	0.74
114.	*Panicum turgidum* Forssk MUH-1839	-	Poaceae	Extract of whole plant is used to treat different diseases like wound healing, throat infection, smallpox	21	18	0.26	0.71
115.	*Pennisetum flaccidum* Griseb. MUH-1840	Fountain grass	Poaceae	Plant parts is used to treat different diseases like fever	33	28	0.35	0.62
116.	*Phragmitis karka* (Retz.) MUH-1841	Babyoon	Poaceae	Roots are cooling and used as antidiabetic	28	21	0.48	0.60
117.	*Poa annua* L. MUH-1842	Grass	Poaceae	Whole plant is used as fodder	27	22	0.41	0.62
118.	*Phalaris minor* L. MUH-1843	Bunch grass	Poaceae	Leaves are dried and made Joshanda used to cure cough, cold and other diseases like dysentery, fever, diarrhea.	23	27	0.36	0.74
119.	*Portulaca quadrifida* L. MUH-1844	Jungle kulfa	Protulacaceae	Extract of whole plant is used treat different diseases like antibacterial, anti-inflammatory	21	18	0.26	0.64
120.	*Phyllanthus niruri* L. MUH-1845	Gale of the wind	Phyllanthaceae	Used to cure liver diseases in the form of powder three times daily, anti-inflammatory, antibacterial, antiseptic, liver diseases, diuretic.	33	28	0.35	0.73
121.	*Polygonum plebeium* L. MUH-1846	Knotweed	Polygonaceae	Extract of plant is used to cure different diseases like tonic, treat pneumonia, fever	28	21	0.48	0.60
122.	*Polygonum aviculare* L. MUH-1847	Weed	Polygonaceae	Rhizome infusion is used for the treatment of diseases like against cough, dysentery, diarrhea.	27	22	0.41	0.62
123.	*Polygonatum multiflora* L. MUH-1848	Soolmoon seal	Polygonaceae	Make a paste of rhizome of plant and used to cure different diseases like dysentery, fever, antiseptic, antibacterial, diarrhea.	23	27	0.36	0.74
124.	*Portulaca oleracea* L. MUH-1849	Zangali Warkhrhay	Portulacaceae	Taken leaves cocked as food and used treatment of different diseases. Leaves also used to cure skin diseases externally.	21	18	0.26	0.64
125.	*Rumex acetosella* L. MUH-1854	Garden sorrel	Polygonaceae	Decoction of aerial parts of plant used to cure different diseases like jaundice, urinary, antiseptic, diuretic	28	21	0.31	0.60
126.	*Rumex dentatus* L. MUH-1855	Toothed duck	Polygonaceae	Root and leaves extract are used to cure skin diseases like wound healing, coetaneous disorder.	26	28	0.25	0.71
127.	*Rumex obtusifolius* L. MUH-1856	Jungle palak	Polygonaceae	Infusions of different plants are used to treat different diseases like kidney diseases, colds, cough, asthma	33	28	0.35	0.63
128.	*Rumex chalepensis* Mill. MUH-1857	Hula	Polygonaceae	Extract of whole plant is used to treat different diseases like diuretic, antiseptic, asthma, colds	28	21	0.48	0.60
129.	*Rumex nepalensis* L. MUH-1858	Dock	Polygonaceae	Infusion of leaves is used treat different diseases like stomach diseases, tonic, diarrhea	27	22	0.41	0.62
130.	*Ranunculus sceleratus* Linn. MUH-1859	Gul-eashrafi	Ranunculaceae	Extract of leaves is effective for asthma and cure tumor	23	27	0.36	0.74
131.	*Ranunculus muricatus* L. MUH-1860	Kar-kandoli	Ranunculaceae	Plant extract is used to cure different diseases like cough, asthma, snake bite, tumor	21	18	0.26	0.62
132.	*Ranunculus arvensis* L. MUH-1861	Corn buttercup	Ranunculaceae	Paste of whole plant is used treat different diseases like wound healing, skin diseases	33	28	0.35	0.64
133.	*Ranunculus laetus* L. MUH-1862	Chambal booti	Ranunculaceae	Paste of fresh leaves applied on wounds	28	21	0.48	0.60
134.	*Solanum surattense* Burm. MUH-1867	Marhaghonay	Solanaceae	Whole plant extract is effective for stomach diseases, cough and fever, chest pain	27	22	0.41	0.62
135.	*Setaria pallidefusca* C.E. Hubb.MUH-1868	Bihari grass	Poaceae	Take seed, grind make flour and used to treat skin diseases.	23	27	0.36	0.74
136.	*Saccharum spontaneum* L. MUH-1869	Kaai	Poaceae	Ach of whole plant mixed with water and used treat different diseases like blood disorders, constipation, liver diseases.	21	18	0.26	0.71
137.	*Setaria glauca* L. MUH-1870	Green foxtail	Poaceae	Flour of plant is used to treat skin diseases, such as chicken pox.	33	28	0.35	0.64
138.	*Sporobolus helvolus* L. MUH-1871	Smut grass	Poaceae	Whole plant is used as fodder	28	21	0.48	0.60
139.	*Silybum marianum* Gaertn. MUH-1872	Kanndyara	Asteraceae	Whole plant extract is used treat different disease, antidiabetic, treat skin diseases, anticancer, tumor,	27	22	0.41	0.62
140.	*Sonchus arvensis* L. MUH-1873	Sowthistle	Asteraceae	The extract of leaves is used to treat cough, asthma and cold. The tea of root is used to treat chest pain and anti-inflammatory	23	27	0.36	0.74
141.	*Sonchus asper* (L.) Hell MUH-1874	spiny Sowthistle	Asteraceae	For enhancing milk, shoots give to domestic animals	21	18	0.26	0.62
142.	*Saussurea costus* L. MUH-1875	Kuth	Asteraceae	Root extract is effective for skin disease	33	28	0.35	0.71
143.	*Solanum nigrum* L. MUH-1876	Katch match	Solanaceae	Leaves are crushed in green condition and used to cure warts on skin.	28	21	0.48	0.60
144.	*Sisymbrium irio* L. MUH-1877	Weed	Brassicaceae	Whole plant dried, crushed, makes powder and used to cure heart diseases.	27	22	0.41	0.62
145.	*Silene conoidea* L. MUH-1878	Pataki	Caryophyllaceae	Root tract is used as wound healing and juice is used to cure skin diseases, wound healing, malarial fever, stomach diseases, headache	23	27	0.36	0.74
146.	*Sophora mollis* L. MUH-1879	Phagan booti	Fabaceae	Powder obtained from seeds is used to cure different diseases including joint diseases, kidney diseases	21	18	0.26	0.73
147.	*Trianthema portulacastrum* L. MUH-1880	Itsit	Aizoaceae	Powder of whole plant is used to treat different blood related diseases diuretic, night blindness, anticancerogenic	28	21	0.31	0.60
148.	*Thalictrum minus* L. MUH-1881	Meadow-rue	Ranunculaceae	Root extract is very effective for different diseases like diuretic, stomach diseases, fever, skin diseases.	26	28	0.25	0.64
149.	*Themeda antheria* News. MUH-1882	Red grass	Poaceae	Powder of whole plant parts is ground and used to treat wounds.	33	28	0.35	0.71
150.	*Tribulus terrestris* L. MUH-1883	Bullhead	Zygophyllaceae	Whole plant extraction is used to treat different diseases like kidney diseases, diuretic, tonic, stomach diseases.	28	21	0.48	0.60
151.	*Trichodesma indicum* L. MUH-1884	Borage	Boraginaceae	Leaf paste is applied on wounds for healing	27	22	0.41	0.62
152.	*Tridax procumbens* L. MUH-1885	Kuthi	Asteraceae	The juice extracted from the leaves is directly applied on wounds, antifungal	23	27	0.36	0.74
153.	*Trifolium repens* L. MUH-1886	White clover	Papilionaceae	Plant infusion is used to treat fever. Root extract is used to cure fever and cough.	21	18	0.26	0.73
154.	*Trifolium dubium* L. MUH-1887	Suckling clover	Papilionaceae	Plant extract with water used to cure fever and cold, constipation, antidiabetic, cancer, arthritis	33	28	0.35	0.75
155.	*Trifolium resupinatum* Linn. MUH-1888	Loosin	Papilionaceae	Fodder for animals	28	21	0.48	0.60
156.	*Trichosanthes anguina* L. MUH-1889	Parul	Cucurbitaceae	Extract of fresh leaves is used to treat skin diseases, diabetes and ulcer, antimicrobial, antidiabetic, diuretic, cure ulcers	27	22	0.41	0.62
157.	*Thymus serpyllum* L. MUH-1890	Wild thyme	Lamiaceae	Take shoot of plant make tea with water and used to cure different diseases like fever, constipation, body pain	23	27	0.36	0.74
158.	*Taraxacum officinale* L. MUH-1891	Hand	Asteraceae	Leaves boiled, make paste with salt and haldi used to cure bones	21	18	0.26	0.71
159.	*Typha elephantina* Pers. MUH-1894	Koondar	Typhaceae	Extract of fresh leaves are used to treat stomach related diseases, dysentery	33	28	0.35	0.74
160.	*Vaccaria hispanica* (Mill.) Rauschert MUH-1899	Masna	Caryophyllaceae	A decoction is used to treat different diseases, menstrual problem, skin problems, breast tumor	28	21	0.48	0.60
161.	*Viola canescens* Wall.ex Roxb. MUH-1900	Banafsha	Violaceae	Take flowers mixed with sugar make kahwa to treat cough, fever, sore throat.	27	22	0.41	0.62
162.	*Vicia sativa* Retz. MUH-1901	-	Papilionaceae	Plant is dried make powder used with water to cure diseases, cure asthma, cough, skin diseases, tonic, diuretic	23	27	0.36	0.74
163.	*Vallaris solanacea* (Roth) O. Kuntze. MUH-1902	Dhudi	Apocynaceae	Paste of whole plant is used to treat different diseases like antimicrobial, antidiabetic, skin infection, wound healing	21	18	0.26	0.63
164.	*Veronica anagallis* L. MUH-903	Hazar booti	Scrophulariaceae	Medicines are used to treat throat diseases.	33	28	0.35	0.72
165.	*Veronica thapsus* L. MUH-1904	-	Scrophulariaceae	Leaves of plant are used to treat different diseases like tonic other skin diseases	28	21	0.48	0.60
166.	*Veronica polita* Fr. MUH-1905	Sriri	Plantaginaceae	Juice or extract of plant is used treat cuts, burns, sore throat infection	27	22	0.41	0.62
167.	*Vicia sativa* L. MUH-1906	_	Papilionaceae	Powder of whole plant is used to treat different diseases like antimicrobial, antioxidant,antidiabetic, diuretic.	23	27	0.36	0.74
168.	*Vicia hirsuta* L. MUH-1907	-	Papilionaceae	Powder of whole plant is used to treat different diseases like diuretic, antidiabetic, antioxidant, antimicrobial	21	18	0.26	0.71
169.	*Vicoa indica* L. MUH-1908	Golden daisy	Asteraceae	Leaves are boiled with water and used orally to treat different diseases like dysentery and other digestive diseases	26	28	0.25	0.64
170.	*Valeriana wallichii* L. MUH-1909	Mushkbala	Valerianaceae	Powder of whole plant is used to treat different diseases like sedative, stomachic, obesity, snake poisoning, nervous disorders and skin diseases.	33	28	0.35	0.71
171.	*Withania somnifera* L. MUH-1910	Dodak	Solanaceae	Make powder of root or fruit and used with milk or honey to cure nervous disorders, ulcers, anti-inflammatory	28	21	0.48	0.60
172.	*Woodfordia fruticosa* (L.) Kurz MUH-1911	Tahvi	Lythraceae	Powder of whole plant is used to treat different diseases like fever, dysentery, toothache	33	28	0.35	0.67
173.	*Xanthium strumarium* L. MUH-1912	Bakhra	Asteraceae	Leaves are crushed and used for curing different diseases like small pox, malarial fever, dysentery and poisons.	28	21	0.48	0.60

### Priority Ranking (PR)

According to the information gathered it is predicted that use of plant for various house cores is common in study area. Extensive use of plant and its products causes reduction in respected abundance of plant species. The priority ranking (PR) analysis determines the abundance status of each ethnobotanically reported plants species. Data was organized into tubular form and destructive order was determined and arranged in six Destructive order is; 4<3<2<1 = 4 number represents the most destructive value, as shown in Table 10. The results depicted that silviculture and clearing of land for agriculture purpose was the key issue of pressure on the herbal flora because due to this phenomenon herbs were cut off or made died due to chemical spray. The fire due to random or deliberate use by farmers to clear unwanted flora from the wild areas was the second important factor affecting the herbaceous flora of the study area. Similar results have been cited by the previous researchers that herbal flora is very sensitive and fragile being easily diminished due to natural or anthropogenic activity [50–52].

**Table 10:** Priority Ranking (PR) of factors apparent as threats to plant diversity on the basis of their level of critical effects in the SMR of district Bhimber (destructive order is; 4<3<2<1 = 4 is highest destructive value).

Factors	Respondent (R1 to R6)						Total	%age	Rank
	R1	R2	R3	R4	R5	R6			
Agricultural use	6	4	5	4	4	6	29	18.83	1^st^
Fuel	2	6	4	2	2	3	19	12.23	4^th^
Fodder	5	3	4	5	2	6	25	16.33	3^rd^
Fire	4	5	5	4	4	5	27	17.53	2^nd^

### Conservation status determination

The current study was primarily focused on documentation of Ethnomedico profiling of herbal flora of Shiwalik Mountaineous Range (SMR) of District Bhimber of AJK. The herbal plants are being small and minute biomass very sensitive for life. These plants are used for different forms by local people like these are as source of ethnobotanical applications. The continuous and incessant cutting or usage by the indigenous communities causes loss of the many of these herbaceous taxa from the study area. In line with the collected data numbers of native plant species from the study are actively used by indigenous people of the area for various uses. Inhabitants of the area relay on natural sources firstly due to lack of resources and secondly due to high cost of mark product. Alongside native inhabitant also believes that herbal medicines are safer for use as compare to pharmaceutical medicines. Extensive use of natural sources is causes serious risk to their abundance percentage. Calculated values represent classification of plants according to risk factors decreasing their abundances. Values determine how respondents of area categorize different threatening parameters for flora of study area. Highest rank of priority ranking (PR) is recorded for consumption of trees for fuel, followed by wood cutting of plants, while lowest is recorded for hedging and thatching. This shows that villagers of study area highly depend upon wood for furniture making, for fuel, in construction and tools making. Whereas fresh parts of trees are used for fodder. This represents key factor that will cause natural flora degradation in study area. Many species like *Aerva sanguinolenta*, *Ajuga bracteosa*, *Boerhavia diffusa*, *Citrullus colocynthis*, *Hyoscyamus niger*, *Solanum surratense*, *Trichodesma indicum and Viola canescens* are declared as threatened species and some of these are endangered. It species is near to extinct from the study area which demands urgent need to conserve these valuable plants. Similar efforts and findings have been cited and recommended for conservation of wild flora of in different areas of Pakistan and world [3, 9, 53–57]. These plants are of high medicinal potential and conservation of these will provide commercial and drug development opportunity for the future generation.

## Conclusion

It is concluded that locals of developing countries are still highly dependent on plant and their sources for various life cores while, urban community is indirectly dependent on plant and their resources. Plants have gained their importance in every core of life. Through recurrent field surveys and interviews from study area it is concluded that almost every individual plant species is somehow used by inhabitants of area. Further quantitative analysis categorized and authenticated the collected data according to their use patterns. Concentrated results were analyzed using various statistical tools to describe the use value and relative importance of cited plant species.

## Recommendations and future threats managements

There is dare need to tree flora of the area because it provides lot of ethnobotanical and folklore herbal therapeutics to cure different ailments in SRM area of District Bhimber, AJK. At a same time where plants and their sources are vital for humans’ plants are also environmental buffers they maintain balances air composition, provides oxygen and some plants (bioengineers) absorbs harmful compounds from soil, maintaining soil pH. Study highly recommends strict rules at governmental level to conserve of most common EB plant species from degradation. There is need to expand the Prime ministers ‘billion’s tree tsunami’ project by involvement of youth in its propagation, cultivation and protection. This will lead towards ‘green revolution’ and make the environment eco-friendly with least pollution impacts as well as timely raining for good agriculture products and crops.
